The article "Estimation of progression of multi-state chronic disease using the Markov model and prevalence pool concept" was retracted in 2009. Reasons: concerns about the data; concerns about the authorship.

# Estimation of progression of multi-state chronic disease using the Markov model and prevalence pool concept

**DOI:** 10.1186/1472-6947-7-34

**Published:** 2007-11-09

**Authors:** Hui-Chuan Shih, Pesus Chou, Chi-Ming Liu, Tao-Hsin Tung

**Affiliations:** 1 Department of Nursing, Kaohsiung Armed Forces General Hospital, Kaohsiung, Taiwan; 2 Community Medicine Research Center and Institute of Public Health, National Yang-Ming University, Taipei, Taiwan; 3 Department of Medical Research and Education, Cheng Hsin Rehabilitation Medical Center, Taipei, Taiwan; 4 Faculty of Public Health, School of Medicine, Fu-Jen Catholic University, Taipei, Taiwan

## Abstract

**Background:**

We propose a simple new method for estimating progression of a chronic disease with multi-state properties by unifying the prevalence pool concept with the Markov process model.

**Methods:**

Estimation of progression rates in the multi-state model is performed using the E-M algorithm. This approach is applied to data on Type 2 diabetes screening.

**Results:**

Good convergence of estimations is demonstrated. In contrast to previous Markov models, the major advantage of our proposed method is that integrating the prevalence pool equation (that the numbers entering the prevalence pool is equal to the number leaving it) into the likelihood function not only simplifies the likelihood function but makes estimation of parameters stable.

**Conclusion:**

This approach may be useful in quantifying the progression of a variety of chronic diseases.

## Background

While the relationship between exposure and outcome is explored in traditional epidemiology, the status of the disease in question is usually expressed as a dichotomous state: disease and non-disease. Categorizing the disease of interest into two states, more often than not, may not only widen the gap between epidemiologists, who are interested in the occurrence of disease, and clinicians, who are concerned with the prognosis of disease, but also limit investigation of the disease progression for the majority of chronic diseases. As a matter of fact, chronic diseases usually have a multi-state property for which a dynamic progression from the early stage to the late stage proceeds under the influence of a range of internal and external risk factors. In order to elucidate the mechanism of disease progression quantifying the multi-state natural history of the disease becomes important in the new era of epidemiology.

Multi-state models are increasingly used to model the progression of chronic diseases [1,2]. Such models are useful for study of both natural history and progression of the related disease [3,4]. Examples include the estimation of transition rates of growth, spread of breast cancer [4], and outcomes of cardiac transplantation [2]. Quantifying the progression of chronic diseases from mild state to advanced state is also relevant to prevention and screening. The multi-state model traditionally associated with chronic diseases has three states: no disease, preclinical but screen-detectable disease, and symptomatic clinical disease.

In the context of screening for chronic diseases, the estimations of progression rates based on mathematical models are usually complicated and computationally intensive. For example, Day and Walter (1984) used screening results of breast cancer to simultaneously estimate false negative cases (cases missed at screen) and the mean sojourn time (the average duration of the screen-detectable phase (PCDP), abbreviated as MST hereafter) based on prevalent screen-detected cases and interval cases (clinical cases occurring between screens) [5]. Duffy et al. (1995) and Chen et al. (1996) also applied stochastic models to estimate parameters of breast tumor progression on the basis of screen-detected and interval cancers. Although these methods had their strengths, some major problems still arose [1,6].

Firstly, time to pre-clinical screen-detectable phase for prevalent screen-detected cases (identified in the first screen) is more uncertain than that for incident screen cases (identified in later screens) because prevalent screen-detected cases are treated as a left-censored mode whereas incident screen-detected cases are classified an interval-censored mode in the context of survival analysis. The latter usually provide more information on the occurrence of event than the former. To simplify the estimation of parameters, previous methods often assume that occurrence of prevalence cases as in exponential distribution which has a property of constant pre-clinical incidence.

Secondly, estimation of parameters in previous methods needs interval cases. However, it may be difficult to obtain interval cases in countries with incomplete registration; one may be concerned with whether estimation of parameters lacking of this information could bias the result. Although a previous study on quantifying the progression of breast cancer demonstrates that estimation of parameters using interval-censored data may yield an unbiased result consistent with those estimates using interval cases it is uncertain whether data on screening for other chronic diseases has the same result. How to treat the missing information on interval cases while relevant parameters are estimated will be considered in this study.

Thirdly, the progression of a multi-state disease may be affected by a set of risk factors or covariates. For example, the onset of Type 2 diabetes may vary by sex, age, obesity and other relevant risk factors. Previous studies on quantifying the progression of chronic diseases either did not take relevant risk factors into account [1,5,6] or considered covariates based on computationally intensive method [7,8].

Fourthly, since certain disease states could not be directly observed, there may be difficulty estimating the model parameters as the models may not be identifiable. This issue is aggravated by a lack of interval cases (cases diagnosed between screens). We find the application of Rothman prevalence pool concept and its extension plus E-M algorithm approach can not only simplify the likelihood function but make estimation of parameters become stable [9]. Missing information on interval cases could be also taken into account.

In this study, a three-state Markov model and an illness-and-death Markov model are proposed to model the progression of multi-state disease natural history. The prevalence pool concept proposed by Rothman is applied to prevalent screen-detected cases to estimate parameters dispensing with the exponential assumptions used in previous studies. To tackle the identifiable problem, an E-M algorithm (Expectation-Maximum likelihood estimate) approach, is proposed to take the prevalence pool equation and its extension to death as expectation equations. Accordingly, these expectation equations in combination with the above two Markov models are then used to estimate relevant parameters. An E-M approach was first advocated by Dempster in 1977 [10]. Since then, an E-M algorithm had been extensively used in handling missing data and dealing with latent variables. The major tenet of this approach is to build up a complete likelihood function as if missing information or latent variables are known. Then, parameters generated from expectation equations are further applied to simplify the likelihood function. This iterative procedure is also used to demonstrate the convergence of parameters.

As above, the aim of this study is to demonstrate how to estimate parameters with respect to multi-state disease progression based on a three-state Markov model plus Rothman prevalence pool concept or an illness-and-death Markov model plus the extension of Rothman prevalence pool concept under the context of an E-M algorithm approach. A Type 2 diabetes screening regime in Taiwan is used as an illustration. The remainder of this study is organized as follows. We first present how to define disease natural history models for Type 2 diabetes, i.e. a three-state Markov model and an illness-and-death Markov model, and then delineate how to apply Rothman prevalence pool concept and an E-M algorithm approach to estimate parameters. Second, an illustration is given using data from a type 2 diabetes screening regime in Taiwan. Third, numerical results and discussion are given respectively.

## Methods

### Markov model specification

#### A three-state Markov model

Suppose the natural history of a chronic disease can be defined by three states, including normal (no detectable disease), asymptomatic (preclinical screen-detectable disease) and symptomatic (clinical disease). The progression rates are expressed as in Figure 1, where *λ*_1 _represents the incidence rate of asymptomatic cases and *λ*_2 _the progression rate from asymptomatic to symptomatic phase. The inverse of *λ*_2 _is the mean sojourn time (MST).

**Figure 1:** A three-state Markov model for a disease natural history.

We assume that there is no possibility of regression from the asymptomatic phase to normal, or from the symptomatic phase to the asymptomatic phase. This assumption has been extensively used in chronic disease screening models [8,11,12].

Given transition parameters *λ*_1 _and *λ*_2_, one can develop transition probabilities for each possible transition during time t on the basis of the forward Kolomogorov equations [13]. The transition probabilities for the above three-state model are expressed in equation (1):

State123123[P11(t)P12(t)P13(t)0P12(t)P23(t)001]=[e−λtλ1(e−λ2t−e−λ1t)λ1−λ21−e−λt−λ1(e−λ2t−e−λ1t)λ1−λ201−e−λ2te−λ2t001]
 MathType@MTEF@5@5@+=feaafiart1ev1aaatCvAUfKttLearuWrP9MDH5MBPbIqV92AaeXatLxBI9gBaebbnrfifHhDYfgasaacPC6xNi=xI8qiVKYPFjYdHaVhbbf9v8qqaqFr0xc9vqFj0dXdbba91qpepeI8k8fiI+fsY=rqGqVepae9pg0db9vqaiVgFr0xfr=xfr=xc9adbaqaaeGacaGaaiaabeqaaeqabiWaaaGcbaqbaeaabiGaaaqaaiabdofatjabdsha0jabdggaHjabdsha0jabdwgaLbqaauaabeqaceaaaeaafaqabeqaeaaaaeaaaeaacWaGaYC=aaaIXaqmaeaacqaIYaGmaeaacWaGaYNaaaaIZaWmaaaabaqbaeqabeGaaaqaauaabeqadeaaaeaacqaIXaqmaeaacqaIYaGmaeaacqaIZaWmaaaabaWaamWaaeaafaqabeWadaaabaGaemiuaa1aaSbaaSqaaiabigdaXiabigdaXaqabaGccqGGOaakcqWG0baDcqGGPaqkaeaacqWGqbaudaWgaaWcbaGaeGymaeJaeGOmaidabeaakiabcIcaOiabdsha0jabcMcaPaqaaiabdcfaqnaaBaaaleaacqaIXaqmcqaIZaWmaeqaaOGaeiikaGIaemiDaqNaeiykaKcabaGaeGimaadabaGaemiuaa1aaSbaaSqaaiabigdaXiabikdaYaqabaGccqGGOaakcqWG0baDcqGGPaqkaeaacqWGqbaudaWgaaWcbaGaeGOmaiJaeG4mamdabeaakiabcIcaOiabdsha0jabcMcaPaqaaiabicdaWaqaaiabicdaWaqaaiabigdaXaaaaiaawUfacaGLDbaaaaaaaaqaaaqaaiabg2da9maadmaabaqbaeqabmWaaaqaaiabdwgaLnaaCaaaleqabaGaeyOeI0ccciGae83UdWMaemiDaqhaaaGcbaqcfa4aaSaaaeaacqWF7oaBdaWgaaqaaiabigdaXaqabaGaeiikaGIaemyzau2aaWbaaeqabaGaeyOeI0Iae83UdW2aaSbaaeaacqaIYaGmaeqaaiabdsha0baacqGHsislcqWGLbqzdaahaaqabeaacqGHsislcqWF7oaBdaWgaaqaaiabigdaXaqabaGaemiDaqhaaiabcMcaPaqaaiab=T7aSnaaBaaabaGaeGymaedabeaacqGHsislcqWF7oaBdaWgaaqaaiabikdaYaqabaaaaaGcbaGaeGymaeJaeyOeI0Iaemyzau2aaWbaaSqabeaacqGHsislcqWF7oaBcqWG0baDaaGccqGHsisljuaGdaWcaaqaaiab=T7aSnaaBaaabaGaeGymaedabeaacqGGOaakcqWGLbqzdaahaaqabeaacqGHsislcqWF7oaBdaWgaaqaaiabikdaYaqabaGaemiDaqhaaiabgkHiTiabdwgaLnaaCaaabeqaaiabgkHiTiab=T7aSnaaBaaabaGaeGymaedabeaacqWG0baDaaGaeiykaKcabaGae83UdW2aaSbaaeaacqaIXaqmaeqaaiabgkHiTiab=T7aSnaaBaaabaGaeGOmaidabeaaaaaakeaacqaIWaamaeaacqaIXaqmcqGHsislcqWGLbqzdaahaaWcbeqaaiabgkHiTiab=T7aSnaaBaaameaacqaIYaGmaeqaaSGaemiDaqhaaaGcbaGaemyzau2aaWbaaSqabeaacqGHsislcqWF7oaBdaWgaaadbaGaeGOmaidabeaaliabdsha0baaaOqaaiabicdaWaqaaiabicdaWaqaaiabigdaXaaaaiaawUfacaGLDbaaaaaaaa@BA3F@

#### An illness-and-death Markov model

When death is taken into account, we further formulate a four-state Markov model as Figure 2. The transition probabilities for a four-state illness-and-death Markov can be derived in a similar manner. The detailed algebra for transition probabilities is given in Appendix A.

**Figure 2:** A four-state illness-and-death Markov model.

### Prevalence pool concept

The concept of the prevalence pool was firstly used by Rothman and Greenland (1998) [9]. Brookmeyer (1995) applied this concept to estimate progression rates associated with HIV and AIDS [14]. It states that, in a steady population, the number of people entering the prevalence pool is balanced by the number exiting from it. That is,

Inflow (to prevalence pool) = outflow (from prevalence pool)

Rothman used this concept to derive the relationship between prevalence and incidence. This concept can be extended to any equilibrium state with respect to disease progression. In the above three-state model, for example, a linear relationship between the asymptomatic and symptomatic phase, in the context of screening, can be defined as follows. The first screen in a screening regime contains prevalent asymptomatic cases. If the total number of subjects attending the screen is N and the prevalence pool (number of asymptomatic phase cases) is P, then the size of population at risk that fed the prevalence pool is N-P. During a very small time interval Δt, the number of subjects who enter the prevalence pool is *λ*_1_Δt (N-P), where *λ*_1 _is the incidence rate of asymptomatic phase. During the same interval Δt, the outflow from the prevalence pool is *λ*_2_Δt P, where *λ*_2 _is the rate of exiting from the prevalence pool, i.e., the hazard rate of surfacing to the symptomatic phase.

According to the above prevalence pool concept, a linear relationship between *λ*_1 _and *λ*_2 _is obtained as follows:

Inflow = *λ*_1_Δt (N-P) = outflow = *λ*_2_Δt P

λ2=N−PP×λ1
 MathType@MTEF@5@5@+=feaafiart1ev1aaatCvAUfKttLearuWrP9MDH5MBPbIqV92AaeXatLxBI9gBaebbnrfifHhDYfgasaacPC6xNi=xI8qiVKYPFjYdHaVhbbf9v8qqaqFr0xc9vqFj0dXdbba91qpepeI8k8fiI+fsY=rqGqVepae9pg0db9vqaiVgFr0xfr=xfr=xc9adbaqaaeGacaGaaiaabeqaaeqabiWaaaGcbaacciGae83UdW2aaSbaaSqaaiabikdaYaqabaGccqGH9aqpjuaGdaWcaaqaaiabd6eaojabgkHiTiabdcfaqbqaaiabdcfaqbaakiabgEna0kab=T7aSnaaBaaaleaacqaIXaqmaeqaaaaa@39F8@

This forms what we will call hereafter the expectation equation. The Markov model in combination with the prevalence pool concept enables us to estimate the parameters using an E-M algorithm approach. In a similar way, the prevalence pool concept can be applied to an illness-and-death model which includes death as an absorbing state.

Taking death into account, we extend the prevalence pool concept to derive the relationship between *λ*_2 _and *λ*_3_. If P asymptomatic phase cases are detected and the follow-up period J is relatively short, the expected symptomatic phase cases (C_E_) if the screen has not taken place is:

C_E _= *λ*_2 _× J × P

The above expression assumes deaths from asymptomatic cases are rare.

Despite early intervention, some asymptomatic cases will progress to symptomatic disease and then to death. Assuming an average time of progression to symptomatic disease midway through the period J, the total number of expected death from symptomatic disease is approximately:

D_E _= *λ*_3 _× J/2 × C_E_

This gives the relationship between *λ*_2 _and *λ*_3_:

λ3=2DEJ2×P×λ2
 MathType@MTEF@5@5@+=feaafiart1ev1aaatCvAUfKttLearuWrP9MDH5MBPbIqV92AaeXatLxBI9gBaebbnrfifHhDYfgasaacPC6xNi=xI8qiVKYPFjYdHaVhbbf9v8qqaqFr0xc9vqFj0dXdbba91qpepeI8k8fiI+fsY=rqGqVepae9pg0db9vqaiVgFr0xfr=xfr=xc9adbaqaaeGacaGaaiaabeqaaeqabiWaaaGcbaacciGae83UdW2aaSbaaSqaaiabiodaZaqabaGccqGH9aqpjuaGdaWcaaqaaiabikdaYiabdseaenaaBaaabaGaemyraueabeaaaeaacqWGkbGsdaahaaqabeaacqaIYaGmaaGaey41aqRaemiuaaLaey41aqRae83UdW2aaSbaaeaacqaIYaGmaeqaaaaaaaa@3E2B@

In a steady population, the relationship between *λ*_1 _and *λ*_3 _via prevalence pool equation (2) is therefore:

λ3=2DEJ2×(N−P)×λ1
 MathType@MTEF@5@5@+=feaafiart1ev1aaatCvAUfKttLearuWrP9MDH5MBPbIqV92AaeXatLxBI9gBaebbnrfifHhDYfgasaacPC6xNi=xI8qiVKYPFjYdHaVhbbf9v8qqaqFr0xc9vqFj0dXdbba91qpepeI8k8fiI+fsY=rqGqVepae9pg0db9vqaiVgFr0xfr=xfr=xc9adbaqaaeGacaGaaiaabeqaaeqabiWaaaGcbaacciGae83UdW2aaSbaaSqaaiabiodaZaqabaGccqGH9aqpjuaGdaWcaaqaaiabikdaYiabdseaenaaBaaabaGaemyraueabeaaaeaacqWGkbGsdaahaaqabeaacqaIYaGmaaGaey41aqRaeiikaGIaemOta4KaeyOeI0IaemiuaaLaeiykaKIaey41aqRae83UdW2aaSbaaeaacqaIXaqmaeqaaaaaaaa@41ED@

### An E-M algorithm approach

The E-M algorithm is an iterative method for estimating parameters in two steps: The E-step (expectation step) and the M-step (maximization step) [10]. Let Y represent the observed data and Z missing data or latent variables (in our case, Z represents subjects who dropped out after the first screen). The E-step augments the observed data Y with the latent data Z. Doing so can simplify the likelihood function in order to obtain a maximum likelihood estimate in the M-step. Formally, we define the E-M algorithm in the same way as Tanner (1996) [15]. Let *λ*^i ^represent the current guess to the mode of observed posterior P(*λ*|Y). The observed data Y includes the first screen (Y_1_), the second screen (Y_2_), and deaths (D). For the sake of brevity, we let Y'_1 _denote a vector including Y_1 _and D. Thus, P (*λ*|Y_2_, Y'_1_, Z) denotes the augmented and simplified posterior distribution and P (Z, Y'_1_|Y_2_, *λ*^i^) denotes the conditional predictive distribution of missing data Z and Y'_1_, conditional on the current guess to the posterior mode.

In the E-step, the computation is as follows:

Q(λ,λi)=∫∫log⁡[P(λ|Z,Y1',Y2)]P(Z,Y1'|λi,Y2)dZdY1'
 MathType@MTEF@5@5@+=feaafiart1ev1aaatCvAUfKttLearuWrP9MDH5MBPbIqV92AaeXatLxBI9gBaebbnrfifHhDYfgasaacPC6xNi=xI8qiVKYPFjYdHaVhbbf9v8qqaqFr0xc9vqFj0dXdbba91qpepeI8k8fiI+fsY=rqGqVepae9pg0db9vqaiVgFr0xfr=xfr=xc9adbaqaaeGacaGaaiaabeqaaeqabiWaaaGcbaGaemyuaeLaeiikaGccciGae83UdWMaeiilaWIae83UdW2aaWbaaSqabeaacqWGPbqAaaGccqGGPaqkcqGH9aqpcqGHRiI8cqGHRiI8cyGGSbaBcqGGVbWBcqGGNbWzcqGGBbWwcqWGqbaucqGGOaakcqWF7oaBcqGG8baFcqWGAbGwcqGGSaalcqWGzbqwdaqhaaWcbaGaeGymaedabaGaei4jaCcaaOGaeiilaWIaemywaK1aaSbaaSqaaiabikdaYaqabaGccqGGPaqkcqGGDbqxcqWGqbaucqGGOaakcqWGAbGwcqGGSaalcqWGzbqwdaqhaaWcbaGaeGymaedabaGaei4jaCcaaOGaeiiFaWNae83UdW2aaWbaaSqabeaacqWGPbqAaaGccqGGSaalcqWGzbqwdaWgaaWcbaGaeGOmaidabeaakiabcMcaPiabdsgaKjabdQfaAjabdsgaKjabdMfaznaaDaaaleaacqaIXaqmaeaacqGGNaWjaaaaaa@65F7@

In the M-step, parameters are estimated by:

∂Q(λ,λi)∂λ|λ=0
 MathType@MTEF@5@5@+=feaafiart1ev1aaatCvAUfKttLearuWrP9MDH5MBPbIqV92AaeXatLxBI9gBaebbnrfifHhDYfgasaacPC6xNi=xI8qiVKYPFjYdHaVhbbf9v8qqaqFr0xc9vqFj0dXdbba91qpepeI8k8fiI+fsY=rqGqVepae9pg0db9vqaiVgFr0xfr=xfr=xc9adbaqaaeGacaGaaiaabeqaaeqabiWaaaGcbaqcfa4aaSaaaeaacqGHciITcqWGrbqucqGGOaakiiGacqWF7oaBcqGGSaalcqWF7oaBdaahaaqabeaacqWGPbqAaaGaeiykaKcabaGaeyOaIyRae83UdWgaaOGaeiiFaW3aaSbaaSqaaiab=T7aSbqabaGccqGH9aqpcqaIWaamaaa@3F41@

In addition to missing data on interval cases, we simplify the likelihood by indirectly estimating parameters via the prevalence pool equation (2) and the illness-death equation (4) using data from Y1'
 MathType@MTEF@5@5@+=feaafiart1ev1aaatCvAUfKttLearuWrP9MDH5MBPbIqV92AaeXatLxBI9gBaebbnrfifHhDYfgasaacPC6xNi=xH8viVGI8Gi=hEeeu0xXdbba9frFj0xb9qqpG0dXdb9aspeI8k8fiI+fsY=rqGqVepae9pg0db9vqaiVgFr0xfr=xfr=xc9adbaqaaeGacaGaaiaabeqaaeqabiWaaaGcbaGaemywaK1aa0baaSqaaiabigdaXaqaaiabcEcaNaaaaaa@2F01@. Instead of estimating *λ*_1 _and *λ*_2 _simultaneously in a three-state Markov model, we augment the observed data and simplify the likelihood function in this study by only estimating *λ*_1 _in the M-step, given the expected *λ*_2_, which is derived from the prevalence pool equation. In other words, we use observed data from the first screen in combination with the prevalence pool equation to simplify the likelihood function based on data from the second screen. A similar procedure is also applied to the illness-and-death Markov model.

Since subjects may attend the first screen but may be lost to follow up we therefore perform one analysis based on complete data only and one estimating missing data in the E-M algorithm.

#### Complete data analysis

For a three-state model, suppose we only have data on two rounds of screening. Let N_1 _and N_2 _represent subjects attending the first screen and the second screen, respectively. The corresponding asymptomatic phase cases in each screen are P_1 _and P_2_, respectively. Let x be the time interval in years between the first and second screen. The likelihood function for data from the second screen is developed using the transition probabilities in (1). The transition probabilities for asymptomatic phase cases and screen negative cases are P_11_(t) and P_12_(t), respectively. Recall that we estimate *λ*_1 _given the expected *λ*_2_, which is estimated on the basis of the prevalence pool equation. For a three-state model, the application of expressions (2) and (5) to this data yield the following E-step computation:

Q(λ1,λ1i)=E((N2−P2)×log⁡[P11(x)]+P2×log⁡[P12(x)])=((N2−P2)×log⁡(e−λ1x)+P2×log⁡[(λ1λ1−E(λ2|λ1i,Y1))×(e−E(λ2|λ1i,Y1)x−e−λ1x)]
 MathType@MTEF@5@5@+=feaafiart1ev1aaatCvAUfKttLearuWrP9MDH5MBPbIqV92AaeXatLxBI9gBaebbnrfifHhDYfgasaacPC6xNi=xI8qiVKYPFjYdHaVhbbf9v8qqaqFr0xc9vqFj0dXdbba91qpepeI8k8fiI+fsY=rqGqVepae9pg0db9vqaiVgFr0xfr=xfr=xc9adbaqaaeGacaGaaiaabeqaaeqabiWaaaGcbaqbaeWabmqaaaqaaiabdgfarjabcIcaOGGaciab=T7aSnaaBaaaleaacqaIXaqmaeqaaOGaeiilaWIae83UdW2aa0baaSqaaiabigdaXaqaaiabdMgaPbaakiabcMcaPiabg2da9iabdweafjabcIcaOiabcIcaOiabd6eaonaaBaaaleaacqaIYaGmaeqaaOGaeyOeI0Iaemiuaa1aaSbaaSqaaiabikdaYaqabaGccqGGPaqkcqGHxdaTcyGGSbaBcqGGVbWBcqGGNbWzcqGGBbWwcqWGqbaudaWgaaWcbaGaeGymaeJaeGymaedabeaakiabcIcaOiabdIha4jabcMcaPiabc2faDjabgUcaRiabdcfaqnaaBaaaleaacqaIYaGmaeqaaOGaey41aqRagiiBaWMaei4Ba8Maei4zaCMaei4waSLaemiuaa1aaSbaaSqaaiabigdaXiabikdaYaqabaGccqGGOaakcqWG4baEcqGGPaqkcqGGDbqxcqqGPaqkaeaacqGH9aqpcqGGOaakcqGGOaakcqWGobGtdaWgaaWcbaGaeGOmaidabeaakiabgkHiTiabdcfaqnaaBaaaleaacqaIYaGmaeqaaOGaeiykaKIaey41aqRagiiBaWMaei4Ba8Maei4zaCMaeiikaGIaemyzau2aaWbaaSqabeaacqGHsislcqWF7oaBdaWgaaadbaGaeGymaedabeaaliabdIha4baakiabcMcaPaqaaiabgUcaRiabdcfaqnaaBaaaleaacqaIYaGmaeqaaOGaey41aqRagiiBaWMaei4Ba8Maei4zaCMaei4waSLaeiikaGscfa4aaSaaaeaacqWF7oaBdaWgaaqaaiabigdaXaqabaaabaGae83UdW2aaSbaaeaacqaIXaqmaeqaaiabgkHiTiabdweafjabcIcaOiab=T7aSnaaBaaabaGaeGOmaidabeaacqGG8baFcqWF7oaBdaqhaaqaaiabigdaXaqaaiabdMgaPbaacqGGSaalcqWGzbqwdaWgaaqaaiabigdaXaqabaGaeiykaKcaaOGaeiykaKIaey41aqRaeiikaGIaemyzau2aaWbaaSqabeaacqGHsislcqWGfbqrcqGGOaakcqWF7oaBdaWgaaadbaGaeGOmaidabeaaliabcYha8jab=T7aSnaaDaaameaacqaIXaqmaeaacqWGPbqAaaWccqGGSaalcqWGzbqwdaWgaaadbaGaeGymaedabeaaliabcMcaPiabdIha4baakiabgkHiTiabdwgaLnaaCaaaleqabaGaeyOeI0Iae83UdW2aaSbaaWqaaiabigdaXaqabaWccqWG4baEaaGccqGGPaqkcqGGDbqxaaaaaa@BC43@

where

E(λ2|λ1i,Y1)=E(λ2|λ1i,P1,N1)=N−P1P1λ1i
 MathType@MTEF@5@5@+=feaafiart1ev1aaatCvAUfKttLearuWrP9MDH5MBPbIqV92AaeXatLxBI9gBaebbnrfifHhDYfgasaacPC6xNi=xI8qiVKYPFjYdHaVhbbf9v8qqaqFr0xc9vqFj0dXdbba91qpepeI8k8fiI+fsY=rqGqVepae9pg0db9vqaiVgFr0xfr=xfr=xc9adbaqaaeGacaGaaiaabeqaaeqabiWaaaGcbaGaemyrauKaeiikaGccciGae83UdW2aaSbaaSqaaiabikdaYaqabaGccqGG8baFcqWF7oaBdaqhaaWcbaGaeGymaedabaGaemyAaKgaaOGaeiilaWIaemywaK1aaSbaaSqaaiabigdaXaqabaGccqGGPaqkcqGH9aqpcqWGfbqrcqGGOaakcqWF7oaBdaWgaaWcbaGaeGOmaidabeaakiabcYha8jab=T7aSnaaDaaaleaacqaIXaqmaeaacqWGPbqAaaGccqGGSaalcqWGqbaudaWgaaWcbaGaeGymaedabeaakiabcYcaSiabd6eaonaaBaaaleaacqaIXaqmaeqaaOGaeiykaKIaeyypa0tcfa4aaSaaaeaacqWGobGtcqGHsislcqWGqbaudaWgaaqaaiabigdaXaqabaaabaGaemiuaa1aaSbaaeaacqaIXaqmaeqaaaaakiab=T7aSnaaDaaaleaacqaIXaqmaeaacqWGPbqAaaaaaa@59C3@

For an illness-and-death model, if the number of deaths in P (= P_1 _+ P_2_) asymptomatic phase cases is denoted as D we used the relationship between *λ*_1 _and *λ*_3 _in expression (4) to obtain the expected *λ*_3 _for simplifying the likelihood function. This is in addition to using the prevalence pool equation to determine the relationship between *λ*_1 _and *λ*_2_. Since time of death is exactly known in principle, an instantaneous rate, dP_24_(*t*), is required. Censored cases, surviving to time *t *are modelled by 1-P_24_(*t*). The computation in the E-step is:

Q(λ1,λ1i)=E[(P2×log⁡[P12(X)]+(N2−P2)×log⁡[P11(X)]+∑i=1Dlog⁡dP24(ui)+∑j=P−DPlog⁡(1−P24(vj))]=(N2−P2)×log⁡(e−λ1t)+P2×log⁡[(λ1X1−E(λ2|λ1i,Y1))×(e−E(λ2|λ1i,Y1)X−e−λ1X)+∑i=1Dlog⁡[(E(λ2|λ1i,Y1)E(λ3|λ1i,Y1,D))×(e−E(λ3|λ1i,Y1,D)t−e−E(λ2|λ1ii,Y1)t)(E(λ2|λ1i,Y1)−E(λ3|λ1i,Y1,D))]+∑j=P−d1Plog⁡(e−E(λ2|λ1i,Y1)t+E(λ2|λ1i,Y1)×e−E(λ3|λ1i,Y1)−e−E(λ2|λ1i,Y1)E(λ2|λ1i,Y1)−E(λ3|λ1i,Y1,D))
 MathType@MTEF@5@5@+=feaafiart1ev1aaatCvAUfKttLearuWrP9MDH5MBPbIqV92AaeXatLxBI9gBaebbnrfifHhDYfgasaacPC6xNi=xI8qiVKYPFjYdHaVhbbf9v8qqaqFr0xc9vqFj0dXdbba91qpepeI8k8fiI+fsY=rqGqVepae9pg0db9vqaiVgFr0xfr=xfr=xc9adbaqaaeGacaGaaiaabeqaaeqabiWaaaGcbaqbaeWabiqaaaqaaiabdgfarjabcIcaOGGaciab=T7aSnaaBaaaleaacqaIXaqmaeqaaOGaeiilaWIae83UdW2aa0baaSqaaiabigdaXaqaaiabdMgaPbaakiabcMcaPaqaauaabaqagiaaaaqaaiabg2da9aqaaiabdweafjabcUfaBjabcIcaOiabdcfaqnaaBaaaleaacqaIYaGmaeqaaOGaey41aqRagiiBaWMaei4Ba8Maei4zaCMaei4waSLaemiuaa1aaSbaaSqaaiabigdaXiabikdaYaqabaGccqGGOaakcqWGybawcqGGPaqkcqGGDbqxcqGHRaWkcqGGOaakcqWGobGtdaWgaaWcbaGaeGOmaidabeaakiabgkHiTiabdcfaqnaaBaaaleaacqaIYaGmaeqaaOGaeiykaKIaey41aqRagiiBaWMaei4Ba8Maei4zaCMaei4waSLaemiuaa1aaSbaaSqaaiabigdaXiabigdaXaqabaGccqGGOaakcqWGybawcqGGPaqkcqGGDbqxaeaaaeaacqGHRaWkdaaeWbqaaiGbcYgaSjabc+gaVjabcEgaNjabdsgaKjabdcfaqnaaBaaaleaacqaIYaGmcqaI0aanaeqaaOGaeiikaGIaemyDau3aaSbaaSqaaiabdMgaPbqabaGccqGGPaqkcqGHRaWkdaaeWbqaaiGbcYgaSjabc+gaVjabcEgaNjabcIcaOiabigdaXiabgkHiTiabdcfaqnaaBaaaleaacqaIYaGmcqaI0aanaeqaaOGaeiikaGIaemODay3aaSbaaSqaaiabdQgaQbqabaGccqGGPaqkcqGGPaqkcqGGDbqxaSqaaiabdQgaQjabg2da9iabdcfaqjabgkHiTiabdseaebqaaiabdcfaqbqdcqGHris5aaWcbaGaemyAaKMaeyypa0JaeGymaedabaGaemiraqeaniabggHiLdaakeaacqGH9aqpaeaacqGGOaakcqWGobGtdaWgaaWcbaGaeGOmaidabeaakiabgkHiTiabdcfaqnaaBaaaleaacqaIYaGmaeqaaOGaeiykaKIaey41aqRagiiBaWMaei4Ba8Maei4zaCMaeiikaGIaemyzau2aaWbaaSqabeaacqGHsislcqWF7oaBdaWgaaadbaGaeGymaedabeaaliabdsha0baakiabcMcaPaqaaaqaaiabgUcaRiabdcfaqnaaBaaaleaacqaIYaGmaeqaaOGaey41aqRagiiBaWMaei4Ba8Maei4zaCMaei4waSLaeiikaGscfa4aaSaaaeaacqWF7oaBdaWgaaqaaiabigdaXaqabaaabaGaemiwaG1aaSbaaeaacqaIXaqmaeqaaiabgkHiTiabdweafjabcIcaOiab=T7aSnaaBaaabaGaeGOmaidabeaacqGG8baFcqWF7oaBdaqhaaqaaiabigdaXaqaaiabdMgaPbaacqGGSaalcqWGzbqwdaWgaaqaaiabigdaXaqabaGaeiykaKcaaOGaeiykaKIaey41aqRaeiikaGIaemyzau2aaWbaaSqabeaacqGHsislcqWGfbqrcqGGOaakcqWF7oaBdaWgaaadbaGaeGOmaidabeaaliabcYha8jab=T7aSnaaDaaameaacqaIXaqmaeaacqWGPbqAaaWccqGGSaalcqWGzbqwdaWgaaadbaGaeGymaedabeaaliabcMcaPiabdIfaybaakiabgkHiTiabdwgaLnaaCaaaleqabaGaeyOeI0Iae83UdW2aaSbaaWqaaiabigdaXaqabaWccqWGybawaaGccqGGPaqkaeaaaeaacqGHRaWkdaaeWbqaaiGbcYgaSjabc+gaVjabcEgaNjabcUfaBjabcIcaOiabdweafjabcIcaOiab=T7aSnaaBaaaleaacqaIYaGmaeqaaOGaeiiFaWNae83UdW2aa0baaSqaaiabigdaXaqaaiabdMgaPbaakiabcYcaSiabdMfaznaaBaaaleaacqaIXaqmaeqaaOGaeiykaKIaemyrauKaeiikaGIae83UdW2aaSbaaSqaaiabiodaZaqabaGccqGG8baFcqWF7oaBdaqhaaWcbaGaeGymaedabaGaemyAaKgaaOGaeiilaWIaemywaK1aaSbaaSqaaiabigdaXaqabaGccqGGSaalcqWGebarcqGGPaqkcqGGPaqkcqGHxdaTjuaGdaWcaaqaaiabcIcaOiabdwgaLnaaCaaabeqaaiabgkHiTiabdweafjabcIcaOiab=T7aSnaaBaaabaGaeG4mamdabeaacqGG8baFcqWF7oaBdaqhaaqaaiabigdaXaqaaiabdMgaPbaacqGGSaalcqWGzbqwdaWgaaqaaiabigdaXaqabaGaeiilaWIaemiraqKaeiykaKIaemiDaqhaaiabgkHiTiabdwgaLnaaCaaabeqaaiabgkHiTiabdweafjabcIcaOiab=T7aSnaaBaaabaGaeGOmaidabeaacqGG8baFcqWF7oaBdaqhaaqaaiabigdaXiabdMgaPbqaaiabdMgaPbaacqGGSaalcqWGzbqwdaWgaaqaaiabigdaXaqabaGaeiykaKIaemiDaqhaaiabcMcaPaqaaiabcIcaOiabdweafjabcIcaOiab=T7aSnaaBaaabaGaeGOmaidabeaacqGG8baFcqWF7oaBdaqhaaqaaiabigdaXaqaaiabdMgaPbaacqGGSaalcqWGzbqwdaWgaaqaaiabigdaXaqabaGaeiykaKIaeyOeI0IaemyrauKaeiikaGIae83UdW2aaSbaaeaacqaIZaWmaeqaaiabcYha8jab=T7aSnaaDaaabaGaeGymaedabaGaemyAaKgaaiabcYcaSiabdMfaznaaBaaabaGaeGymaedabeaacqGGSaalcqWGebarcqGGPaqkcqGGPaqkaaGccqGGDbqxaSqaaiabdMgaPjabg2da9iabigdaXaqaaiabdseaebqdcqGHris5aaGcbaaabaGaey4kaSYaaabCaeaacyGGSbaBcqGGVbWBcqGGNbWzcqGGOaakcqWGLbqzdaahaaWcbeqaaiabgkHiTiabdweafjabcIcaOiab=T7aSnaaBaaameaacqaIYaGmaeqaaSGaeiiFaWNae83UdW2aa0baaWqaaiabigdaXaqaaiabdMgaPbaaliabcYcaSiabdMfaznaaBaaameaacqaIXaqmaeqaaSGaeiykaKIaemiDaqhaaOGaey4kaScaleaacqWGQbGAcqGH9aqpcqWGqbaucqGHsislcqWGKbazdaWgaaadbaGaeGymaedabeaaaSqaaiabdcfaqbqdcqGHris5aOGaemyrauKaeiikaGIae83UdW2aaSbaaSqaaiabikdaYaqabaGccqGG8baFcqWF7oaBdaqhaaWcbaGaeGymaedabaGaemyAaKgaaOGaeiilaWIaemywaK1aaSbaaSqaaiabigdaXaqabaGccqGGPaqkcqGHxdaTjuaGdaWcaaqaaiabdwgaLnaaCaaabeqaaiabgkHiTiabdweafjabcIcaOiab=T7aSnaaBaaabaGaeG4mamdabeaacqGG8baFcqWF7oaBdaqhaaqaaiabigdaXaqaaiabdMgaPbaacqGGSaalcqWGzbqwdaWgaaqaaiabigdaXaqabaGaeiykaKcaaiabgkHiTiabdwgaLnaaCaaabeqaaiabgkHiTiabdweafjabcIcaOiab=T7aSnaaBaaabaGaeGOmaidabeaacqGG8baFcqWF7oaBdaqhaaqaaiabigdaXaqaaiabdMgaPbaacqGGSaalcqWGzbqwdaWgaaqaaiabigdaXaqabaGaeiykaKcaaaqaaiabdweafjabcIcaOiab=T7aSnaaBaaabaGaeGOmaidabeaacqGG8baFcqWF7oaBdaqhaaqaaiabigdaXaqaaiabdMgaPbaacqGGSaalcqWGzbqwdaWgaaqaaiabigdaXaqabaGaeiykaKIaeyOeI0IaemyrauKaeiikaGIae83UdW2aaSbaaeaacqaIZaWmaeqaaiabcYha8jab=T7aSnaaDaaabaGaeGymaedabaGaemyAaKgaaiabcYcaSiabdMfaznaaBaaabaGaeGymaedabeaacqGGSaalcqWGebarcqGGPaqkaaGccqGGPaqkaaaaaaaa@DD8E@

where P = P_1 _+ P_2_

D is the number of deaths

P-D is the number of censored cases

u_i_: exact death time

v_j_: censored time

Note that *λ*_2 _and *λ*_3 _are repeatedly estimated by

E(λ2|λ1i,Y1)=E(λ2|λ1i,P1,N1)=N−P1P1λ1iE(λ3|λ1i,Y1,D)=E(λ3|λ1i,P1,N1,D)=2DJ2×(N1−P1)×λ1
 MathType@MTEF@5@5@+=feaafiart1ev1aaatCvAUfKttLearuWrP9MDH5MBPbIqV92AaeXatLxBI9gBaebbnrfifHhDYfgasaacPC6xNi=xI8qiVKYPFjYdHaVhbbf9v8qqaqFr0xc9vqFj0dXdbba91qpepeI8k8fiI+fsY=rqGqVepae9pg0db9vqaiVgFr0xfr=xfr=xc9adbaqaaeGacaGaaiaabeqaaeqabiWaaaGcbaqbaeaabiqaaaqaaiabdweafjabcIcaOGGaciab=T7aSnaaBaaaleaacqaIYaGmaeqaaOGaeiiFaWNae83UdW2aa0baaSqaaiabigdaXaqaaiabdMgaPbaakiabcYcaSiabdMfaznaaBaaaleaacqaIXaqmaeqaaOGaeiykaKIaeyypa0JaemyrauKaeiikaGIae83UdW2aaSbaaSqaaiabikdaYaqabaGccqGG8baFcqWF7oaBdaqhaaWcbaGaeGymaedabaGaemyAaKgaaOGaeiilaWIaemiuaa1aaSbaaSqaaiabigdaXaqabaGccqGGSaalcqWGobGtdaWgaaWcbaGaeGymaedabeaakiabcMcaPiabg2da9KqbaoaalaaabaGaemOta4KaeyOeI0Iaemiuaa1aaSbaaeaacqaIXaqmaeqaaaqaaiabdcfaqnaaBaaabaGaeGymaedabeaaaaGccqWF7oaBdaqhaaWcbaGaeGymaedabaGaemyAaKgaaaGcbaGaemyrauKaeiikaGIae83UdW2aaSbaaSqaaiabiodaZaqabaGccqGG8baFcqWF7oaBdaqhaaWcbaGaeGymaedabaGaemyAaKgaaOGaeiilaWIaemywaK1aaSbaaSqaaiabigdaXaqabaGccqGGSaalcqWGebarcqGGPaqkcqGH9aqpcqWGfbqrcqGGOaaktCvAUfeBSjuyZL2yd9gzLbvyNv2CaeHbuLwBLnhiov2DGi1BTfMBaGabaiaa+T7adaWgaaWcbaGaeG4mamdabeaakiabcYha8jab=T7aSnaaDaaaleaacqaIXaqmaeaacqWGPbqAaaGccqGGSaalcqWGqbaudaWgaaWcbaGaeGymaedabeaakiabcYcaSiabd6eaonaaBaaaleaacqaIXaqmaeqaaOGaeiilaWIaemiraqKaeiykaKIaeyypa0tcfa4aaSaaaeaacqaIYaGmcqWGebaraeaacqWGkbGsdaahaaqabeaacqaIYaGmaaGaey41aqRaeiikaGIaemOta40aaSbaaeaacqaIXaqmaeqaaiabgkHiTiabdcfaqnaaBaaabaGaeGymaedabeaacqGGPaqkcqGHxdaTcqWF7oaBdaWgaaqaaiabigdaXaqabaaaaaaaaaa@9F91@

In the M-step, *λ*_1 _is estimated iteratively by equation (6).

#### Missing data analysis

As stated earlier, some subjects drop out after the first screen. We also use the E-M algorithm to estimate parameters taking this missing information into account. Following the principle of handling missing data proposed by Longford et al. (2000) in diaries of alcohol consumption, E-M algorithm and multiple imputations are used to handle missing data on interval cases [16]. The procedure is described as follows. If there are W dropouts after the first screen, these subjects could have been in three possible states, normal, asymptomatic phase or symptomatic phase, with respective numbers, W_1_, W_2_, and W_3_, between the first screen and second screen. The W follows a multinomial distribution with the corresponding probabilities: P_11_(x), P_12_(x), and P_13_(X) for W_1_, W_2_, and W_3_, given a total of subjects W. The expected values for the corresponding three states are calculated as:

*μ*_*i *_= *W *× *P*_1*i*_(*X*), *i *= 1, 2 and 3

Computation in the E-step is now:

Q(λ1,λ1i)=E((N2−P2+W1)×log⁡[P11(X)]+(P2+W2)×log⁡[P12(X)]+W3×log⁡[P13(X)]))=((N2−P2+μ1)×log⁡(e−λ1x)+(P2+μ2)×log⁡[(λ1λ1−E(λ2|λ1i,Y1)×(e−E(λ2|λ1i,Y1)x−e−λ1x)]+(μ3×log⁡[1−e−λ1x−(λ1λ1−E(λ2|λ1i,Y1))×(e−E(λ2|λ1i,Y1)x−e−λ1x)])
 MathType@MTEF@5@5@+=feaafiart1ev1aaatCvAUfKttLearuWrP9MDH5MBPbIqV92AaeXatLxBI9gBaebbnrfifHhDYfgasaacPC6xNi=xI8qiVKYPFjYdHaVhbbf9v8qqaqFr0xc9vqFj0dXdbba91qpepeI8k8fiI+fsY=rqGqVepae9pg0db9vqaiVgFr0xfr=xfr=xc9adbaqaaeGacaGaaiaabeqaaeqabiWaaaGcbaqbaeaabiqaaaqaaiabdgfarjabcIcaOGGaciab=T7aSnaaBaaaleaacqaIXaqmcqGGSaalaeqaaOGae83UdW2aa0baaSqaaiabigdaXaqaaiabdMgaPbaakiabcMcaPaqaauaabaqafiaaaaqaaiabg2da9aqaaiabdweafjabcIcaOiabcIcaOiabd6eaonaaBaaaleaacqaIYaGmaeqaaOGaeyOeI0Iaemiuaa1aaSbaaSqaaiabikdaYaqabaGccqGHRaWkcqWGxbWvdaWgaaWcbaGaeGymaedabeaakiabcMcaPiabgEna0kGbcYgaSjabc+gaVjabcEgaNjabcUfaBjabdcfaqnaaBaaaleaacqaIXaqmcqaIXaqmaeqaaOGaeiikaGIaemiwaGLaeiykaKIaeiyxa0fabaaabaGaey4kaSIaeiikaGIaemiuaa1aaSbaaSqaaiabikdaYaqabaGccqGHRaWkcqWGxbWvdaWgaaWcbaGaeGOmaidabeaakiabcMcaPiabgEna0kGbcYgaSjabc+gaVjabcEgaNjabcUfaBjabdcfaqnaaBaaaleaacqaIXaqmcqaIYaGmaeqaaOGaeiikaGIaemiwaGLaeiykaKIaeiyxa0Laey4kaSIaem4vaC1aaSbaaSqaaiabiodaZaqabaGccqGHxdaTcyGGSbaBcqGGVbWBcqGGNbWzcqGGBbWwcqWGqbaudaWgaaWcbaGaeGymaeJaeG4mamdabeaakiabcIcaOiabdIfayjabcMcaPiabc2faDjabcMcaPiabcMcaPaqaaiabg2da9aqaaiabbIcaOiabbIcaOGqaciab+5eaonaaBaaaleaacqqGYaGmaeqaaOGaeyOeI0Iaemiuaa1aaSbaaSqaaiabikdaYaqabaGccqGHRaWkcqWF8oqBdaWgaaWcbaGaeGymaedabeaakiabcMcaPiabgEna0kGbcYgaSjabc+gaVjabcEgaNjabcIcaOiabdwgaLnaaCaaaleqabaGaeyOeI0Iae83UdW2aaSbaaWqaaiabigdaXaqabaWccqWG4baEaaGccqGGPaqkaeaaaeaacqGHRaWkcqGGOaakcqWGqbaudaWgaaWcbaGaeGOmaidabeaakiabgUcaRiab=X7aTnaaBaaaleaacqaIYaGmaeqaaOGaeiykaKIaey41aqRagiiBaWMaei4Ba8Maei4zaCMaei4waSLaeiikaGscfa4aaSaaaeaacqWF7oaBdaWgaaqaaiabigdaXaqabaaabaGae83UdW2aaSbaaeaaieaacqqFXaqmaeqaaiabgkHiTiabdweafjabcIcaOiab=T7aSnaaBaaabaGaeGOmaidabeaacqGG8baFcqWF7oaBdaqhaaqaaiabigdaXaqaaiabdMgaPbaacqGGSaalcqWGzbqwdaWgaaqaaiabigdaXaqabaGaeiykaKcaaOGaey41aqRaeiikaGIaemyzau2aaWbaaSqabeaacqGHsislcqWGfbqrcqGGOaakcqWF7oaBdaWgaaadbaGaeGOmaidabeaaliabcYha8jab=T7aSnaaDaaameaacqaIXaqmaeaacqWGPbqAaaWccqGGSaalcqWGzbqwdaWgaaadbaGaeGymaedabeaaliabcMcaPiabdIha4baakiabgkHiTiabdwgaLnaaCaaaleqabaGaeyOeI0Iae83UdW2aaSbaaWqaaiabigdaXaqabaWccqWG4baEaaGccqGGPaqkcqGGDbqxaeaaaeaacqGHRaWkcqqGOaakcqWF8oqBdaWgaaWcbaGaee4mamdabeaakiabgEna0kGbcYgaSjabc+gaVjabcEgaNjabcUfaBjabigdaXiabgkHiTiabdwgaLnaaCaaaleqabaGaeyOeI0Iae83UdW2aaSbaaWqaaiabigdaXaqabaWccqWG4baEaaGccqGHsislcqGGOaakjuaGdaWcaaqaaiab=T7aSnaaBaaabaGaeGymaedabeaaaeaacqWF7oaBdaWgaaqaaiabigdaXaqabaGaeyOeI0IaemyrauKaeiikaGIae83UdW2aaSbaaeaacqaIYaGmaeqaaiabcYha8jab=T7aSnaaDaaabaGaeGymaedabaGaemyAaKgaaiabcYcaSiabdMfaznaaBaaabaGaeGymaedabeaacqGGPaqkaaGccqGGPaqkcqGHxdaTcqGGOaakcqWGLbqzdaahaaWcbeqaaiabgkHiTiabdweafjabcIcaOiab=T7aSnaaBaaameaacqaIYaGmaeqaaSGaeiiFaWNae83UdW2aa0baaWqaaiabigdaXaqaaiabdMgaPbaaliabcYcaSiabdMfaznaaBaaameaacqaIXaqmaeqaaSGaeiykaKIaemiEaGhaaOGaeyOeI0Iaemyzau2aaWbaaSqabeaacqGHsislcqWF7oaBdaWgaaadbaGaeGymaedabeaaliabdIha4baakiabcMcaPiabc2faDjabcMcaPaaaaaaaaa@2C14@

As above, *λ*_1 _is estimated in the M-step by iteration according to the score function as in the complete data analysis. *λ*_2 _is estimated by iteration using the prevalence pool equation. Estimation of parameters

The program for estimating parameters in M-step is written using Mathematica software version 3.0 [17]. The details of iteration between E-step and M-step are as follows. For the three-state Markov model, *λ*_2 _^(0) ^is first guessed and an estimate of *λ*_1 _^(1) ^is obtained on the basis of (6) and (7).

1. Substitution of *λ *_1 _^(1) ^into the prevalence pool equation (2)

yields a new estimate of *λ *_2 _^(1)^

2. Repeat procedures (1) and (2) until *λ*_1 _and *λ*_2 _converge to four decimal points.

A similar procedure is applied to the illness-and-death model.

### An E-M approach taking covariates into account

The E-M algorithm approach can be extended to estimate parameters making allowance for covariates affecting the progression rates. For instance, suppose preclinical incidence (*λ*_1_) increases with age. Two approaches are used to consider this problem. The first is based on a stratified analysis by age, in which two separate E-M estimations are performed in age groups < 50 and 50+. This yields independent estimates of *λ*_1 _and *λ*_2 _for each age group.

Another method to take covariates into account is the use of exponential hazard regression to model the effects of covariates on the relevant progression rates. Let age, dichotomized by two groups as in the above, be considered as a covariate and labeled by x = 1 for age over 50 years and x = 0 otherwise. The exponential hazard regression with respect to the preclinical incidence rates for the two groups is written as follows:

*λ*_12 _= *λ*_11 _exp (*β*_1_*x*)

The progression rates from the asymptomatic to symptomatic phase for two age groups (*λ*_21 _and *λ*_22_) are estimated using the prevalence pool equation stratified by age. Thus we have a single E-step estimating both *λ*_11 _and *β*, and two M-steps at each iteration.

### Variance estimation

As *λ*_1 _is estimated given *λ*_2 _in the three-state model, and given *λ*_2 _and *λ*_3 _in the illness-and-death model, the variance of *λ*_1 _calculated through the inverse of the second derivative of the likelihood function in the expression (7) or (8) will be underestimated in that this is a conditional, rather than an unconditional, estimate. Details of calculating the unconditional variance for *λ*_1_, *λ*_2 _and *λ*_3 _are given in Appendix B.

## Results

The above method is applied to data on Type 2 diabetes screening for subjects aged over 30 years in Taiwan. The details of the study design and execution have been described in full elsewhere [18]. In brief, three rounds of screening were conducted between 1987 and 1995 with an approximate 4-year inter-screening interval. All overnight fasting and 2 h serum and plasma samples (preserved with EDTA and NaF) were collected and kept frozen (-20°C) until analysis. Fasting plasma glucose concentrations were determined using the hexokmase-glucose-6-phosphate dehydrogenase method with a glucose (HK) reagent ldt (Gilford, Oberlin, OH).

Three-fixed cohorts, 1987, 1991 and 1995, were identified according to when subjects attended their first screen. Because few subjects attended the third screen in 1995 as a first screen, we excluded them from analysis. Subjects who did not take the oral glucose tolerance test (OGTT) were also excluded from the analysis. For the 1987 cohort, 66 (8.9%) of the 678 patients tested had asymptomatic Type 2 diabetes. Among 678 subjects, only 237 (35%) subjects attended the second screening (1991) with complete information on OGTT test. Of these, 10 had newly diagnosed asymptomatic Type 2 diabetes. For the 1991 cohort, 39 (8.2%) of the 475 subjects were detected as having asymptomatic Type 2 diabetes at the time of the first screening. Thus, a total of 105 (39 + 66) asymptomatic Type 2 diabetes cases were ascertained at first screen. To ascertain deaths from Type 2 diabetes (ICD code 250), the above 115 asymptomatic Type 2 diabetes patients were followed until Dec 1997. Of the 115 subjects, 8 had died of Type 2 diabetes. The average follow-up was 8.29 years. Table 1 summarizes the observed transitions and corresponding transition probabilities used in the three-state Markov model and the illness-and-death Markov model.

**Table 1:** Descriptive results of early detection of Type 2 diabetes for two fixed cohorts in Puli, Taiwan

**Number of Transition**		**Type of Transition**	**Transition probability**
(1) First screen			
Asymptomatic			
Type 2 diabetes	105	(1 → 2, age at first screen(A))	P_12_(A)
Negative	1114	(1 → 1, age at first screen(A))	P_11_(A)
Total	1219		

(2) Second screen			
Asymptomatic			
Type 2 diabetes	10	(1 → 2, 4 year)	P_12_(X)
Negative	227	(1 → 1, 4 year)	P_11_(X)
Total	237		
Death	8	(1 → 4, time to death(t))	dP_21_(X)

Table 2 shows the estimated results for a three-state Markov model. After three iterations the convergence of *λ*_1 _and *λ*_2 _was met. We started from the guessed value of λ2(0)
 MathType@MTEF@5@5@+=feaafiart1ev1aaatCvAUfKttLearuWrP9MDH5MBPbIqV92AaeXatLxBI9gBaebbnrfifHhDYfgasaacPC6xNi=xH8viVGI8Gi=hEeeu0xXdbba9frFj0xb9qqpG0dXdb9aspeI8k8fiI+fsY=rqGqVepae9pg0db9vqaiVgFr0xfr=xfr=xc9adbaqaaeGacaGaaiaabeqaaeqabiWaaaGcbaacciGae83UdW2aa0baaSqaaiabikdaYaqaaiabcIcaOiabicdaWiabcMcaPaaaaaa@314D@ equal to 11.76% using the inverse of the ratio of prevalence (8.6136%), estimated by cases at first screen, to the incidence rate (1.0132%) estimated by cases at second screen divided by 987 person-years. Given this rate, λ1(1)
 MathType@MTEF@5@5@+=feaafiart1ev1aaatCvAUfKttLearuWrP9MDH5MBPbIqV92AaeXatLxBI9gBaebbnrfifHhDYfgasaacPC6xNi=xH8viVGI8Gi=hEeeu0xXdbba9frFj0xb9qqpG0dXdb9aspeI8k8fiI+fsY=rqGqVepae9pg0db9vqaiVgFr0xfr=xfr=xc9adbaqaaeGacaGaaiaabeqaaeqabiWaaaGcbaacciGae83UdW2aa0baaSqaaiabigdaXaqaaiabcIcaOiabigdaXiabcMcaPaaaaaa@314D@ was estimated as 0.107594 according to the above method. The prevalence pool equation was further applied to estimate λ2(1)
 MathType@MTEF@5@5@+=feaafiart1ev1aaatCvAUfKttLearuWrP9MDH5MBPbIqV92AaeXatLxBI9gBaebbnrfifHhDYfgasaacPC6xNi=xH8viVGI8Gi=hEeeu0xXdbba9frFj0xb9qqpG0dXdb9aspeI8k8fiI+fsY=rqGqVepae9pg0db9vqaiVgFr0xfr=xfr=xc9adbaqaaeGacaGaaiaabeqaaeqabiWaaaGcbaacciGae83UdW2aa0baaSqaaiabikdaYaqaaiabcIcaOiabigdaXiabcMcaPaaaaaa@314F@ as: 11.4152%(=(N−P)×0.107594P=(1219−105)×0.107594105)
 MathType@MTEF@5@5@+=feaafiart1ev1aaatCvAUfKttLearuWrP9MDH5MBPbIqV92AaeXatLxBI9gBaebbnrfifHhDYfgasaacPC6xNi=xH8viVGI8Gi=hEeeu0xXdbba9frFj0xb9qqpG0dXdb9aspeI8k8fiI+fsY=rqGqVepae9pg0db9vqaiVgFr0xfr=xfr=xc9adbaqaaeGacaGaaiaabeqaaeqabiWaaaGcbaGaeGymaeJaeGymaeJaeiOla4IaeGinaqJaeGymaeJaeGynauJaeGOmaiJaeiyjauIaeiikaGIaeyypa0tcfa4aaSaaaeaacqGGOaakcqWGobGtcqGHsislcqWGqbaucqGGPaqkcqGHxdaTcqaIWaamcqGGUaGlcqaIXaqmcqaIWaamcqaI3aWncqaI1aqncqaI5aqocqaI0aanaeaacqWGqbauaaGccqGH9aqpjuaGdaWcaaqaaiabcIcaOiabigdaXiabikdaYiabigdaXiabiMda5iabgkHiTiabigdaXiabicdaWiabiwda1iabcMcaPiabgEna0kabicdaWiabc6caUiabigdaXiabicdaWiabiEda3iabiwda1iabiMda5iabisda0aqaaiabigdaXiabicdaWiabiwda1aaakiabcMcaPaaa@5DDC@. The annual preclinical incidence rate of *λ*_1 _was estimated as 1.08% (95% CI: 0.45%–2.58%). The annual progression rate of *λ*_2 _was estimated as 11% (95% CI: 0.06–0.21). The inverse of *λ*_2 _yielded approximately 8 years of mean sojourn time (MST). The stratified analysis in combination with E-M algorithm gave 1.51% (95% CI: 0.49%–4.70%) and 0.75% (95% CI: 0.19%–3.00%) of annual preclinical incidence rate of (*λ*_1_), and 9% and 19% of annual progression rate of *λ*_2 _for aged over 50 years and aged under 50 years, respectively (Table 2). Subjects aged over 50 years had a two-fold risk of occurrence of asymptomatic Type 2 diabetes compared with those aged under 50 years. The approach based on exponential hazard regression yielded similar results (Table 3). The rate ratio of *λ*_1 _for aged over 50 years against aged under 50 years was estimated as 2.01 (e^0.70^). The estimates of *λ*_1 _and *λ*_2 _based on exponential regression were very close to those based on stratified analysis in Table 2.

**Table 2:** The E-M iteration results for a three-state Markov model

	***Parameter***	
*Iteration*	*λ*_1_*(95% CI)*	*λ*_2_*(95% CI)*

Overall		
-----	----------	0.1176
1	0.0108	0.1141
2	0.0108	0.1141
3	0.0108	0.1142
	(0.0045~0.0258)	(0.0614~0.2122)

≥ 50 yrs		
-----	---------	0.1176
1	0.0151	0.0926
2	0.0151	0.0926
3	0.0151	0.0926
	(0.0049~0.0470)	(0.0416~0.2062)

<50 yrs		
-----	----------	0.1176
1	0.0075	0.1934
2	0.0075	0.1933
3	0.0075	0.1933
	0.0075	0.1933
	(0.0019~0.0300)	(0.0732~0.5099)

*λ*_1_:normal → asymptomatic *λ*_2_:asymptomatic → symptomatic

**Table 3:** The E-M iteration results for a Three-state Markov model taking age as a covariate in proportional hazard regression model

	**Parameter**				
	
*Iteration*	*β*	*(≥ 50 yrs)*		*(< 50 yrs)*	
	
	*(95% CI)*	*λ*_11_	*λ*_21_	*λ*_12_	*λ*_22_
-----	---------	----------	0.0926	----------	0.1934
1	0.7008	0.0151	0.0926	0.0075	0.1933
2	0.7008	0.0151	0.0926	0.0075	0.1933
3	0.7008	0.0151	0.0926	0.0075	0.1933
	(0.0681~7.2133)				

*λ*_11 _&*λ*_12_:normal → asymptomatic.

*λ*_21 _&*λ*_22_:asymptomatic → symptomatic

Table 4 shows the estimated results taking the missing data on interval cases into account. These estimates were very similar to those not allowing for missing data in Table 2. This suggests that missing information did not affect the point estimates of *λ*_1 _and *λ*_2 _although the confidence intervals allowing for missing data were narrower than those obtained without taking missing information into account.

**Table 4:** The E-M iteration results for a Three-state Markov model taking missing data on interval cases into account

	Parameter	
	
*Iteration*	*λ*_1_*(95% CI*	*λ*_2_*(95% CI)*
Overall		

0	0.0103	0.1089
1	0.0104	0.1107
5	0.0107	0.1135
6	0.0107	0.1135
	(0.0064~0.0180)	(0.0786~0.1639)

≥ 50 yrs		
0	0.0151	0.1176
1	0.0151	0.0926
11	0.0151	0.0926
12	0.0151	0.0926
	(0.0078~0.0294)	(0.0579~0.1482)

< 50 yrs		
0	0.0075	0.1176
1	0.0075	0.1934
15	0.0075	0.1933
16	0.0075	0.1933
	(0.0029~0.0192)	(0.0993~0.3761)

*λ*_1_:normal → asymptomatic. *λ*_2_:asymptomatic → symptomatic

The estimated results for the four-state illness-and-death model are presented in Table 5. As in the three-state Markov model, λ2(0)
 MathType@MTEF@5@5@+=feaafiart1ev1aaatCvAUfKttLearuWrP9MDH5MBPbIqV92AaeXatLxBI9gBaebbnrfifHhDYfgasaacPC6xNi=xH8viVGI8Gi=hEeeu0xXdbba9frFj0xb9qqpG0dXdb9aspeI8k8fiI+fsY=rqGqVepae9pg0db9vqaiVgFr0xfr=xfr=xc9adbaqaaeGacaGaaiaabeqaaeqabiWaaaGcbaacciGae83UdW2aa0baaSqaaiabikdaYaqaaiabcIcaOiabicdaWiabcMcaPaaaaaa@314D@ and λ3(0)
 MathType@MTEF@5@5@+=feaafiart1ev1aaatCvAUfKttLearuWrP9MDH5MBPbIqV92AaeXatLxBI9gBaebbnrfifHhDYfgasaacPC6xNi=xH8viVGI8Gi=hEeeu0xXdbba9frFj0xb9qqpG0dXdb9aspeI8k8fiI+fsY=rqGqVepae9pg0db9vqaiVgFr0xfr=xfr=xc9adbaqaaeGacaGaaiaabeqaaeqabiWaaaGcbaacciGae83UdW2aa0baaSqaaiabiodaZaqaaiabcIcaOiabicdaWiabcMcaPaaaaaa@314F@ were first guessed and λ1(1)
 MathType@MTEF@5@5@+=feaafiart1ev1aaatCvAUfKttLearuWrP9MDH5MBPbIqV92AaeXatLxBI9gBaebbnrfifHhDYfgasaacPC6xNi=xH8viVGI8Gi=hEeeu0xXdbba9frFj0xb9qqpG0dXdb9aspeI8k8fiI+fsY=rqGqVepae9pg0db9vqaiVgFr0xfr=xfr=xc9adbaqaaeGacaGaaiaabeqaaeqabiWaaaGcbaacciGae83UdW2aa0baaSqaaiabigdaXaqaaiabcIcaOiabigdaXiabcMcaPaaaaaa@314D@ was estimated as 0.0107594. Again, λ2(1)
 MathType@MTEF@5@5@+=feaafiart1ev1aaatCvAUfKttLearuWrP9MDH5MBPbIqV92AaeXatLxBI9gBaebbnrfifHhDYfgasaacPC6xNi=xH8viVGI8Gi=hEeeu0xXdbba9frFj0xb9qqpG0dXdb9aspeI8k8fiI+fsY=rqGqVepae9pg0db9vqaiVgFr0xfr=xfr=xc9adbaqaaeGacaGaaiaabeqaaeqabiWaaaGcbaacciGae83UdW2aa0baaSqaaiabikdaYaqaaiabcIcaOiabigdaXiabcMcaPaaaaaa@314F@ was estimated on the basis of the prevalence pool equation.

λ3(1)(=2×8(8.29)2×(1219−105)×0.0107594)
 MathType@MTEF@5@5@+=feaafiart1ev1aaatCvAUfKttLearuWrP9MDH5MBPbIqV92AaeXatLxBI9gBaebbnrfifHhDYfgasaacPC6xNi=xH8viVGI8Gi=hEeeu0xXdbba9frFj0xb9qqpG0dXdb9aspeI8k8fiI+fsY=rqGqVepae9pg0db9vqaiVgFr0xfr=xfr=xc9adbaqaaeGacaGaaiaabeqaaeqabiWaaaGcbaacciGae83UdW2aa0baaSqaaiabiodaZaqaaiabcIcaOiabigdaXiabcMcaPaaakiabcIcaOiabg2da9KqbaoaalaaabaGaeGOmaiJaey41aqRaeGioaGdabaGaeiikaGIaeGioaGJaeiOla4IaeGOmaiJaeGyoaKJaeiykaKYaaWbaaeqabaGaeGOmaidaaiabgEna0kabcIcaOiabigdaXiabikdaYiabigdaXiabiMda5iabgkHiTiabigdaXiabicdaWiabiwda1iabcMcaPiabgEna0kabicdaWiabc6caUiabicdaWiabigdaXiabicdaWiabiEda3iabiwda1iabiMda5iabisda0aaakiabcMcaPaaa@5559@ was estimated via the illness-and-death equation. The estimates of *λ*_1 _and *λ*_2 _were close to those obtained from Table 2. The annual rate of death from Type 2 diabetes was estimated as 1.94%. Results from the stratified analysis also showed that older subjects had an approximately four-fold for risk for death from Type 2 diabetes compared with younger subjects.

**Table 5:** The E-M iteration results for the illness-and-death Markov model

	*Parameter*		
	
*Iteration*	*λ*_1_*(95% CI)*	*λ*_2_*(95% CI)*	*λ*_3_*(95% CI)*
Overall			
-----	---------	0.1176	0.0100
1	0.0108	0.1142	0.0194
2	0.0108	0.1142	0.0194
3	0.0108	0.1142	0.0194
	(0.0045~0.0258)	(0.0614~0.2122)	(0.0063~0.0600)

≥ 50 yrs			
-----	---------	0.1176	0.0100
1	0.0151	0.0926	0.0258
2	0.0151	0.0926	0.0258
3	0.0151	0.0926	0.0258
	(0.0049~0.0469)	(0.0416~0.2062)	(0.0064~0.1033)

< 50 yrs			
-----	--------	0.1176	0.0100
1	0.0075	0.1934	0.0068
2	0.0075	0.1933	0.0068
3	0.0075	0.1933	0.0068
	(0.0019~0.0300)	(0.0725~0.5149)	(0.0005~0.0906)

*λ*_1_:normal → asymptomatic ; *λ*_2_:asymptomatic → symptomatic.

*λ*_3_:symptomatic → death of Type 2 diabetes

## Discussion

Markov chain models are a natural approach to take when modeling the transitions of patients between discrete health states over time. Welton and Ades (2005) provided a unified Bayesian approach to propagation of uncertainty from both fully and partially observed event history data to Markov model parameters [19]. In this study, we propose a new approach, based on the E-M algorithm, to estimate the progression of a multi-state chronic disease using the prevalence pool concept and Markov process models. From the methodological viewpoint, one limitation of our approach is that the prevalence pool concept is only appropriate in a population where rates of disease are assumed to be at a steady state and this assumption may not necessarily apply to diabetes today, given the recent rapid increase in incidence of diabetes in some countries today. Furthermore, our population data sample was restricted only to subjects with complete OGTT data, and thus some selection bias might have occurred. Finally, Type 2 diabetes occurs in older populations for whom death is a significant competing risk; both subjects without disease and those with asymptomatic disease may also die from other causes. We did not have enough data information to formulate a more complete model which includes competing mortality. Further studies are needed to explore how competing risks could influence the parameters of natural history.

Nevertheless, there are several strengths of this approach. Firstly, it is not as computationally intensive as a single stage estimation using the traditional Markov model. The parameter estimation is simplified by integrating the illness and death equation into the likelihood function. The traditional three-state model usually estimates *λ*_1 _and *λ*_2 _simultaneously using a full likelihood function. Therefore, the likelihood function in the traditional method is more complicated than that in the present study. In addition, simultaneous estimation of *λ*_1 _and *λ*_2 _may encounter a collinearity problem due to a high correlation between two parameters. This phenomenon may be observed when there is no data on interval cases, which are sometimes unavailable for unregistered conditions such as Type 2 diabetes. That is, it is hard to disaggregate the overall rate into distinct rates for each individual state transition if we have little information on the intermediate states. Moreover, our E-M algorithm approach can also take account of missing data on interval cases. This has not been considered in previous studies when interval cases were not available.

Secondly, the previous parametric method of modeling the first screen data usually required the assumption of constant pre-clinical incidence over all ages, which may be unrealistic. Our approach can dispense with this assumption and can estimate *λ*_1 _in the E-step using an age-specific prevalence rate.

Thirdly, results from our approach can be readily applied to design of studies. Suppose we wish to design a randomized trial of screening in this population. We estimate *λ*_1_, *λ*_2 _and *λ*_3 _as 0.011, 0.114 and 0.019 (Table 5). From equation (2) we would expect the prevalence at first screen to be *λ*_1_/(*λ*_1 _+ *λ*_2_) = 88/1000. These cases could be expected to have 5-year cumulative death rate, that is, D_E _= *λ*_3 _× 5/2 × *λ*_2 _× 5 = 0.027. Clinical type 2 diabetes arising spontaneously would be expected to have a different mortality rate *λ*_4 _from those arising from progression of asymptomatic screen-detected cases. Mortality from spontaneous symptomatic cases can be estimated from the case series of Chen et al. (1999) in which there were 131/766 = 0.17 deaths in an average follow-up of 3.5 years [20]. This gives an estimate for *λ*_4 _of 0.054. We would therefore expect deaths from spontaneous interval cases of

∫05λ1e−λ1t∫05−tλ2e−λ2v∫05−t−vλ4e−λ4ududvdt=(1−e−5λ1)−λ1λ4(e−5λ1−e−5λ2)(λ4−λ2)(λ2−λ1)+λ1λ2(e−5λ1−e−5λ4)(λ4−λ2)(λ4−λ1)
 MathType@MTEF@5@5@+=feaafiart1ev1aaatCvAUfKttLearuWrP9MDH5MBPbIqV92AaeXatLxBI9gBaebbnrfifHhDYfgasaacPC6xNi=xI8qiVKYPFjYdHaVhbbf9v8qqaqFr0xc9vqFj0dXdbba91qpepeI8k8fiI+fsY=rqGqVepae9pg0db9vqaiVgFr0xfr=xfr=xc9adbaqaaeGacaGaaiaabeqaaeqabiWaaaGcbaqbaeaabiqaaaqaamaapedabaacciGae83UdW2aaSbaaSqaaiabigdaXaqabaGccqWGLbqzdaahaaWcbeqaaiabgkHiTiab=T7aSnaaBaaameaacqaIXaqmaeqaaSGaemiDaqhaaaqaaiabicdaWaqaaiabiwda1aqdcqGHRiI8aOWaa8qmaeaacqWF7oaBdaWgaaWcbaGaeGOmaidabeaaaeaacqaIWaamaeaacqaI1aqncqGHsislcqWG0baDa0Gaey4kIipakiabdwgaLnaaCaaaleqabaGaeyOeI0Iae83UdW2aaSbaaWqaaiabikdaYaqabaWccqWG2bGDaaGcdaWdXaqaaiab=T7aSnaaBaaaleaacqaI0aanaeqaaOGaemyzau2aaWbaaSqabeaacqGHsislcqWF7oaBdaWgaaadbaGaeGinaqdabeaaliabdwha1baaaeaacqaIWaamaeaacqaI1aqncqGHsislcqWG0baDcqGHsislcqWG2bGDa0Gaey4kIipakiabdsgaKjabdwha1jabdsgaKjabdAha2jabdsgaKjabdsha0bqaaiabg2da9iabcIcaOiabigdaXiabgkHiTiabdwgaLnaaCaaaleqabaGaeyOeI0IaeGynauJae83UdW2aaSbaaWqaaiabigdaXaqabaaaaOGaeiykaKIaeyOeI0scfa4aaSaaaeaacqWF7oaBdaWgaaqaaiabigdaXaqabaGae83UdW2aaSbaaeaacqaI0aanaeqaaiabcIcaOiabdwgaLnaaCaaabeqaaiabgkHiTiabiwda1iab=T7aSnaaBaaabaGaeGymaedabeaaaaGaeyOeI0Iaemyzau2aaWbaaeqabaGaeyOeI0IaeGynauJae83UdW2aaSbaaeaacqaIYaGmaeqaaaaacqGGPaqkaeaacqGGOaakcqWF7oaBdaWgaaqaaiabisda0aqabaGaeyOeI0Iae83UdW2aaSbaaeaacqaIYaGmaeqaaiabcMcaPiabcIcaOiab=T7aSnaaBaaabaGaeGOmaidabeaacqGHsislcqWF7oaBdaWgaaqaaiabigdaXaqabaGaeiykaKcaaOGaey4kaSscfa4aaSaaaeaacqWF7oaBdaWgaaqaaiabigdaXaqabaGae83UdW2aaSbaaeaacqaIYaGmaeqaaiabcIcaOiabdwgaLnaaCaaabeqaaiabgkHiTiabiwda1iab=T7aSnaaBaaabaGaeGymaedabeaaaaGaeyOeI0Iaemyzau2aaWbaaeqabaGaeyOeI0IaeGynauJae83UdW2aaSbaaeaacqaI0aanaeqaaaaacqGGPaqkaeaacqGGOaakcqWF7oaBdaWgaaqaaiabisda0aqabaGaeyOeI0Iae83UdW2aaSbaaeaacqaIYaGmaeqaaiabcMcaPiabcIcaOiab=T7aSnaaBaaabaGaeGinaqdabeaacqGHsislcqWF7oaBdaWgaaqaaiabigdaXaqabaGaeiykaKcaaaaaaaa@BBB0@

after a little algebra. Substituting for *λ*_1_, *λ*_2_, and *λ*_4_, the above is equal to 0.0011. We would therefore expect, per thousand screened and then followed up for 5 years, 88 × 0.027 + 912 × 0.0011, i.e., 3.4 deaths per thousand.

In an unscreened control group, one would expect the number of death to be the number from progression of those in the prevalence pool plus the number from new cases arising, i.e.,

88×∫05λ2e−λ2t∫05−tλ4e−λ4vdvdt+912×0.0011
 MathType@MTEF@5@5@+=feaafiart1ev1aaatCvAUfKttLearuWrP9MDH5MBPbIqV92AaeXatLxBI9gBaebbnrfifHhDYfgasaacPC6xNi=xI8qiVKYPFjYdHaVhbbf9v8qqaqFr0xc9vqFj0dXdbba91qpepeI8k8fiI+fsY=rqGqVepae9pg0db9vqaiVgFr0xfr=xfr=xc9adbaqaaeGacaGaaiaabeqaaeqabiWaaaGcbaGaeGioaGJaeGioaGJaey41aq7aa8qmaeaaiiGacqWF7oaBdaWgaaWcbaGaeGOmaidabeaakiabdwgaLnaaCaaaleqabaGaeyOeI0Iae83UdW2aaSbaaWqaaiabikdaYaqabaWccqWG0baDaaaabaGaeGimaadabaGaeGynaudaniabgUIiYdGcdaWdXaqaaiab=T7aSnaaBaaaleaacqaI0aanaeqaaaqaaiabicdaWaqaaiabiwda1iabgkHiTiabdsha0bqdcqGHRiI8aOGaemyzau2aaWbaaSqabeaacqGHsislcqWF7oaBdaWgaaadbaGaeGinaqdabeaaliabdAha2baakiabdsgaKjabdAha2jabdsgaKjabdsha0jabgUcaRiabiMda5iabigdaXiabikdaYiabgEna0kabicdaWiabc6caUiabicdaWiabicdaWiabigdaXiabigdaXaaa@5ED3@

=88×(1−e−λ25−λ2(e−5λ2−e−5λ4)(λ2−λ4))+1.0032
 MathType@MTEF@5@5@+=feaafiart1ev1aaatCvAUfKttLearuWrP9MDH5MBPbIqV92AaeXatLxBI9gBaebbnrfifHhDYfgasaacPC6xNi=xI8qiVKYPFjYdHaVhbbf9v8qqaqFr0xc9vqFj0dXdbba91qpepeI8k8fiI+fsY=rqGqVepae9pg0db9vqaiVgFr0xfr=xfr=xc9adbaqaaeGacaGaaiaabeqaaeqabiWaaaGcbaGaeyypa0JaeGioaGJaeGioaGJaey41aqRaeiikaGIaeGymaeJaeyOeI0Iaemyzau2aaWbaaSqabeaacqGHsisliiGacqWF7oaBdaWgaaadbaGaeGOmaidabeaaliabiwda1aaakiabgkHiTmaalaaabaGae83UdW2aaSbaaSqaaiabikdaYaqabaGccqGGOaakcqWGLbqzdaahaaWcbeqaaiabgkHiTiabiwda1iab=T7aSnaaBaaameaacqaIYaGmaeqaaaaakiabgkHiTiabdwgaLnaaCaaaleqabaGaeyOeI0IaeGynauJae83UdW2aaSbaaWqaaiabisda0aqabaaaaOGaeiykaKcabaGaeiikaGIae83UdW2aaSbaaSqaaiabikdaYaqabaGccqGHsislcqWF7oaBdaWgaaWcbaGaeGinaqdabeaakiabcMcaPaaacqGGPaqkcqGHRaWkcqaIXaqmcqGGUaGlcqaIWaamcqaIWaamcqaIZaWmcqaIYaGmaaa@5CD7@

= 88 × 0.0586 = 6.2 per thousand.

To have 50% power to detect the difference between the 5-year death of 6.2 and 3.4 as significant, we would need 1,718 subjects per arm.

The above assumes 100% compliance and perfect sensitivity. To cope with some anticipated non-compliance and imperfect sensitivity, we might expect to have, say, 70% of the 88 per thousand in the prevalence pool. The remaining 30% would then arise as interval cases, and the expected death rate in the study arm over 5 years would be 62 × 0.027 + 26 × 0.0586 + 912 × 0.0011 = 4.2 per thousand. For 90% power in this case, we would require 5,177 subjects per arm.

This method can also be adapted to take into account covariates affecting the progression rates of the disease by use of stratified analysis or proportional hazard regression model. Although the only covariate used in this study was age, the approach can accommodate a set of covariates if necessary. Also, the E-M algorithm used in this study was extended to estimate missing information on interval cases.

To check whether parameters estimated from the proposed method were valid, a goodness of fit test was performed to check the adequacy of models. As Table 6 shows, there were no significant differences between the observed and expected rates for an illness-and-death Markov model. A similar finding was observed for the three-state model (data not shown). This suggests a good fit of the model for empirical data.

**Table 6:** Results for the goodness of fit for the illness-and-death Markov model

*Parameter*	*Observed*	*Expected*	*Residual*
Overall			
Negative of first screen	1114	1102	11.998
Positive of first screen	105	117	-11.998
Negative of second screen	227	227.02	-0.016
Positive of second screen	10	8.04	1.9569
Death	8	6.07	1.9254
χ^2 ^= 2.4473 P = 0.2941			
≥ 50 yrs			
Negative of first screen	496	483.471	12.5289
Positive of first screen	81	93.529	-12.5289
Negative of second screen	96	96.011	-0.0109
Positive of second screen	6	4.995	1.0046
Death	7	5.447	1.5534
χ^2 ^= 2.6481 P = 0.2661			
< 50 yrs			
Negative of first screen	618	617.084	0.9157
Positive of first screen	24	24.916	-0.9157
Negative of second screen	131	131.007	0.0073
Positive of second screen	4	2.775	1.2246
Death	1	0.728	0.2715
χ^2 ^= 0.6765 P = 0.7130			

## Conclusion

In conclusion, a simple E-M algorithm approach using the prevalence pool concept and its extension in conjunction with the Markov model was proposed to estimate parameters pertaining to progression rates of chronic disease. This approach may be useful to quantify the multi-state natural history of certain chronic diseases and to evaluate disease screening strategies.

## Competing interests

The author(s) declare that they have no competing interests.

## Authors' contributions

HC and CM participated in the design of the study and performed the statistical analysis. P and TH conceived of the study and participated in its design and coordination. All authors read and approved the final manuscript.

## Appendix A Transition probabilities in the four state model

The transition probabilities for an illness-and-death model are:

P=12341234[P11(t)P12(t)P13(t)P14(t)0P22(t)P23(t)P24(t)00P33(t)P34(t)0001]
 MathType@MTEF@5@5@+=feaafiart1ev1aaatCvAUfKttLearuWrP9MDH5MBPbIqV92AaeXatLxBI9gBaebbnrfifHhDYfgasaacPC6xNi=xI8qiVKYPFjYdHaVhbbf9v8qqaqFr0xc9vqFj0dXdbba91qpepeI8k8fiI+fsY=rqGqVepae9pg0db9vqaiVgFr0xfr=xfr=xc9adbaqaaeGacaGaaiaabeqaaeqabiWaaaGcbaGaemiuaaLaeyypa0tbaeqabiqaaaqaauaabeqabuaaaaqaaaqaaiadacik8daaigdaXaqaaiadaci++daaikdaYaqaaiadacixbaaaiodaZaqaaiadacijdaaaisda0aaaaeaafaqabeqacaaabaqbaeqabqqaaaaabaGaeGymaedabaGaeGOmaidabaGaeG4mamdabaGaeGinaqdaaaqaamaadmaabaqbaeqabqabaaaaaeaacqWGqbaudaWgaaWcbaGaeGymaeJaeGymaedabeaakiabcIcaOiabdsha0jabcMcaPaqaaiabdcfaqnaaBaaaleaacqaIXaqmcqaIYaGmaeqaaOGaeiikaGIaemiDaqNaeiykaKcabaGaemiuaa1aaSbaaSqaaiabigdaXiabiodaZaqabaGccqGGOaakcqWG0baDcqGGPaqkaeaacqWGqbaudaWgaaWcbaGaeGymaeJaeGinaqdabeaakiabcIcaOiabdsha0jabcMcaPaqaaiabicdaWaqaaiabdcfaqnaaBaaaleaacqaIYaGmcqaIYaGmaeqaaOGaeiikaGIaemiDaqNaeiykaKcabaGaemiuaa1aaSbaaSqaaiabikdaYiabiodaZaqabaGccqGGOaakcqWG0baDcqGGPaqkaeaacqWGqbaudaWgaaWcbaGaeGOmaiJaeGinaqdabeaakiabcIcaOiabdsha0jabcMcaPaqaaiabicdaWaqaaiabicdaWaqaaiabdcfaqnaaBaaaleaacqaIZaWmcqaIZaWmaeqaaOGaeiikaGIaemiDaqNaeiykaKcabaGaemiuaa1aaSbaaSqaaiabiodaZiabisda0aqabaGccqGGOaakcqWG0baDcqGGPaqkaeaacqaIWaamaeaacqaIWaamaeaacqaIWaamaeaacqaIXaqmaaaacaGLBbGaayzxaaaaaaaaaaa@801C@

where states 1, 2, 3 and 4 represent no disease, asymptomatic disease, symptomatic disease and death, respectively, and:

P11(t)=e−λ1tP12(t)=λ1(e−λ1tλ2−λ1+e−λ2tλ1−λ2)P13(t)=λ1λ2(e−λ1t(λ1−λ2)(λ1−λ3)−e−λ2t(λ1−λ2)(λ2−λ3)−e−λ3t(λ1−λ3)(λ3−λ2)P14(t)=1−λ1λ2λ3(e−λ1tλ1(λ1−λ2)(λ1−λ3)+e−λ2tλ2(λ1−λ2)(λ2−λ3)+e−λ3tλ3(λ1−λ3)(λ3−λ2)P22(t)=e−λ2tP23(t)=λ2(e−λ2tλ3−λ2+e−λ3tλ2−λ3)P24(t)=1+λ3e−λ2tλ2−λ3−λ2e−λ3tλ2−λ3P33(t)=e−λ3tP34(t)=1−e−λ3t
 MathType@MTEF@5@5@+=feaafiart1ev1aaatCvAUfKttLearuWrP9MDH5MBPbIqV92AaeXatLxBI9gBaebbnrfifHhDYfgasaacPC6xNi=xI8qiVKYPFjYdHaVhbbf9v8qqaqFr0xc9vqFj0dXdbba91qpepeI8k8fiI+fsY=rqGqVepae9pg0db9vqaiVgFr0xfr=xfr=xc9adbaqaaeGacaGaaiaabeqaaeqabiWaaaGcbaqbaeaabOWaaaaaaeaacqWGqbaudaWgaaWcbaGaeGymaeJaeGymaedabeaakiabcIcaOiabdsha0jabcMcaPaqaaiabg2da9aqaaiabdwgaLnaaCaaaleqabaaccaGae8NeI0ccciGae43UdW2aaSbaaWqaaiabigdaXaqabaWccqWG0baDaaaakeaacqWGqbaudaWgaaWcbaGaeGymaeJaeGOmaidabeaakiabcIcaOiabdsha0jabcMcaPaqaaiabg2da9aqaaiab+T7aSnaaBaaaleaacqaIXaqmaeqaaOGaeiikaGscfa4aaSaaaeaacqWGLbqzdaahaaqabeaacqWFsislcqGF7oaBdaWgaaqaaiabigdaXaqabaGaemiDaqhaaaqaaiab+T7aSnaaBaaabaGaeGOmaidabeaacqGHsislcqGF7oaBdaWgaaqaaiabigdaXaqabaaaaOGaey4kaSscfa4aaSaaaeaacqWGLbqzdaahaaqabeaacqWFsislcqGF7oaBdaWgaaqaaiabikdaYaqabaGaemiDaqhaaaqaaiab+T7aSnaaBaaabaGaeGymaedabeaacqWFsislcqGF7oaBdaWgaaqaaiabikdaYaqabaaaaOGaeiykaKcabaGaemiuaa1aaSbaaSqaaiabigdaXiabiodaZaqabaGccqGGOaakcqWG0baDcqGGPaqkaeaacqGH9aqpaeaacqGF7oaBdaWgaaWcbaGaeGymaedabeaakiab+T7aSnaaBaaaleaacqaIYaGmaeqaaOGaeiikaGscfa4aaSaaaeaacqWGLbqzdaahaaqabeaacqWFsislcqGF7oaBdaWgaaqaaiabigdaXaqabaGaemiDaqhaaaqaamXvP5wqSXMqHnxAJn0BKvguHDwzZbqegqvATv2CG4uz3bIuV1wyUbaceaGaa0hkaiab+T7aSnaaBaaabaGaa0xmaaqabaGae8NeI0Iae43UdW2aaSbaaeaacaqFYaaabeaacaqFPaGaa0hkaiab+T7aSnaaBaaabaGaeGymaedabeaacqWFsislcaqF7oWaaSbaaeaacqaIZaWmaeqaaiabcMcaPaaakiab=jHiTKqbaoaalaaabaGaemyzau2aaWbaaeqabaGae8NeI0Iae43UdW2aaSbaaeaacqaIYaGmaeqaaiabdsha0baaaeaacaqFOaGae43UdW2aaSbaaeaacaqFXaaabeaacqWFsislcqGF7oaBdaWgaaqaaiaa9jdaaeqaaiaa9LcacaqFOaGae43UdW2aaSbaaeaacqaIYaGmaeqaaiab=jHiTiab+T7aSnaaBaaabaGaeG4mamdabeaacqGGPaqkaaGccqWFsisljuaGdaWcaaqaaiabdwgaLnaaCaaabeqaaiab=jHiTiab+T7aSnaaBaaabaGaeG4mamdabeaacqWG0baDaaaabaGaeiikaGIae43UdW2aaSbaaeaacqaIXaqmaeqaaiab=jHiTiab+T7aSnaaBaaabaGaeG4mamdabeaacqGGPaqkcqGGOaakcqGF7oaBdaWgaaqaaiabiodaZaqabaGaeyOeI0Iae43UdW2aaSbaaeaacqaIYaGmaeqaaiabcMcaPaaaaOqaaiabdcfaqnaaBaaaleaacqaIXaqmcqaI0aanaeqaaOGaeiikaGIaemiDaqNaeiykaKcabaGaeyypa0dabaGaeGymaeJaeyOeI0Iae43UdW2aaSbaaSqaaiabigdaXaqabaGccqGF7oaBdaWgaaWcbaGaa0NmaaqabaGccqGF7oaBdaWgaaWcbaGaa03maaqabaGccaqFOaqcfa4aaSaaaeaacqWGLbqzdaahaaqabeaacqWFsislcqGF7oaBdaWgaaqaaiabigdaXaqabaGaemiDaqhaaaqaaiab+T7aSnaaBaaabaGaeGymaedabeaacqGGOaakcqGF7oaBdaWgaaqaaiabigdaXaqabaGae8NeI0Iae43UdW2aaSbaaeaacqaIYaGmaeqaaiabcMcaPiabcIcaOiab+T7aSnaaBaaabaGaeGymaedabeaacqWFsislcqGF7oaBdaWgaaqaaiabiodaZaqabaGaeiykaKcaaOGaey4kaSscfa4aaSaaaeaacqWGLbqzdaahaaqabeaacqWFsislcqGF7oaBdaWgaaqaaiabikdaYaqabaGaemiDaqhaaaqaaiab+T7aSnaaBaaabaGaeGOmaidabeaacqGGOaakcqGF7oaBdaWgaaqaaiabigdaXaqabaGae8NeI0Iae43UdW2aaSbaaeaacqaIYaGmaeqaaiabcMcaPiabcIcaOiab+T7aSnaaBaaabaGaeGOmaidabeaacqWFsislcqGF7oaBdaWgaaqaaiabiodaZaqabaGaeiykaKcaaaGcbaaabaaabaGaey4kaSscfa4aaSaaaeaacqWGLbqzdaahaaqabeaacqWFsislcqGF7oaBdaWgaaqaaiabiodaZaqabaGaemiDaqhaaaqaaiab+T7aSnaaBaaabaGaeG4mamdabeaacqGGOaakcqGF7oaBdaWgaaqaaiabigdaXaqabaGae8NeI0Iae43UdW2aaSbaaeaacqaIZaWmaeqaaiabcMcaPiabcIcaOiab+T7aSnaaBaaabaGaeG4mamdabeaacqGHsislcqGF7oaBdaWgaaqaaiabikdaYaqabaGaeiykaKcaaaGcbaGaemiuaa1aaSbaaSqaaiabikdaYiabikdaYaqabaGccqGGOaakcqWG0baDcqGGPaqkaeaacqGH9aqpaeaacqWGLbqzdaahaaWcbeqaaiabgkHiTiab+T7aSnaaBaaameaacqaIYaGmaeqaaSGaemiDaqhaaaGcbaGaemiuaa1aaSbaaSqaaiabikdaYiabiodaZaqabaGccqGGOaakcqWG0baDcqGGPaqkaeaacqGH9aqpaeaacqGF7oaBdaWgaaWcbaGaeGOmaidabeaakiabcIcaOKqbaoaalaaabaGaemyzau2aaWbaaeqabaGae8NeI0Iae43UdW2aaSbaaeaacqaIYaGmaeqaaiabdsha0baaaeaacqGF7oaBdaWgaaqaaiabiodaZaqabaGaeyOeI0Iae43UdW2aaSbaaeaacqaIYaGmaeqaaaaakiabgUcaRKqbaoaalaaabaGaemyzau2aaWbaaeqabaGae8NeI0Iae43UdW2aaSbaaeaacqaIZaWmaeqaaiabdsha0baaaeaacqGF7oaBdaWgaaqaaiabikdaYaqabaGae8NeI0Iae43UdW2aaSbaaeaacqaIZaWmaeqaaaaakiabcMcaPaqaaiabdcfaqnaaBaaaleaacqaIYaGmcqaI0aanaeqaaOGaeiikaGIaemiDaqNaeiykaKcabaGaeyypa0dabaGaeGymaeJaey4kaSscfa4aaSaaaeaacqGF7oaBdaWgaaqaaiabiodaZaqabaGaemyzau2aaWbaaeqabaGae8NeI0Iae43UdW2aaSbaaeaacqaIYaGmaeqaaiabdsha0baaaeaacqGF7oaBdaWgaaqaaiabikdaYaqabaGae8NeI0Iae43UdW2aaSbaaeaacqaIZaWmaeqaaaaakiab=jHiTKqbaoaalaaabaGae43UdW2aaSbaaeaacqaIYaGmaeqaaiabdwgaLnaaCaaabeqaaiab=jHiTiab+T7aSnaaBaaabaGaeG4mamdabeaacqWG0baDaaaabaGae43UdW2aaSbaaeaacqaIYaGmaeqaaiab=jHiTiab+T7aSnaaBaaabaGaeG4mamdabeaaaaaakeaacqWGqbaudaWgaaWcbaGaeG4mamJaeG4mamdabeaakiabcIcaOiabdsha0jabcMcaPaqaaiabg2da9aqaaiabdwgaLnaaCaaaleqabaGae8NeI0Iae43UdW2aaSbaaWqaaiabiodaZaqabaWccqWG0baDaaaakeaacqWGqbaudaWgaaWcbaGaeG4mamJaeGinaqdabeaakiabcIcaOiabdsha0jabcMcaPaqaaiabg2da9aqaaiabigdaXiabgkHiTiabdwgaLnaaCaaaleqabaGae8NeI0Iae43UdW2aaSbaaWqaaiabiodaZaqabaWccqWG0baDaaaaaaaa@A4C5@

## Appendix B

### B.1 The three-state Markov model

Two parameters, *λ*_1 _and *λ*_2_, were estimated in this model. As stated in the text, the variance of *λ*_1 _was a conditional rather than unconditional estimate. In this case, we should re-calculate the unconditional variance of *λ*_1 _as follows:

*Var*(*λ*_1_) = *Var*(*E*(*λ*_1 _| *λ*_2_) + *E*(*Var*(*λ*_1 _| *λ*_2_)

If the asymptotic theory held, E(Var(*λ*_1_|*λ*_2_)) can be assumed to be equal to the observed Var (*λ*_1_|*λ*_2_), which was obtained from the inverse of the second derivative of the likelihood function given the estimates of *λ*_1 _and *λ*_2 _in Table 2.

The first component via the prevalence pool equation in (B.1) was:

Var(E(λ1|λ2)=Var(PN−P×λ2)=(PN−P)2Var(λ2)
 MathType@MTEF@5@5@+=feaafiart1ev1aaatCvAUfKttLearuWrP9MDH5MBPbIqV92AaeXatLxBI9gBaebbnrfifHhDYfgasaacPC6xNi=xI8qiVKYPFjYdHaVhbbf9v8qqaqFr0xc9vqFj0dXdbba91qpepeI8k8fiI+fsY=rqGqVepae9pg0db9vqaiVgFr0xfr=xfr=xc9adbaqaaeGacaGaaiaabeqaaeqabiWaaaGcbaGaemOvayLaemyyaeMaemOCaiNaeiikaGIaemyrauKaeiikaGccciGae83UdW2aaSbaaSqaaiabigdaXaqabaGccqGG8baFcqWF7oaBdaWgaaWcbaGaeGOmaidabeaakiabcMcaPiabg2da9iabdAfawjabdggaHjabdkhaYjabcIcaOKqbaoaalaaabaGaemiuaafabaGaemOta4KaeyOeI0IaemiuaafaaOGaey41aqRae83UdW2aaSbaaSqaaiabikdaYaqabaGccqGGPaqkcqGH9aqpcqGGOaakjuaGdaWcaaqaaiabdcfaqbqaaiabd6eaojabgkHiTiabdcfaqbaakiabcMcaPmaaCaaaleqabaGaeGOmaidaaOGaemOvayLaemyyaeMaemOCaiNaeiikaGIae83UdW2aaSbaaSqaaiabikdaYaqabaGccqGGPaqkaaa@5CE5@

where P and N are numbers of positive cases and attendants.

Given P and N, an unconditional variance of *λ*_2 _is needed to calculate Var(E(*λ*_1_|*λ*_2_)). However, it is very difficult to obtain unconditional variance of *λ*_2 _unless one has other external data. We used an approximation method to calculate an unconditional variance of *λ*_2 _as follows. Suppose the occurrence of asymptomatic phase cases follows a Poisson distribution, the likelihood function based on the second screen data in Table 1 is:

L(λ1')=(1−e−λ1'×4)10(e−λ1'×4)227
 MathType@MTEF@5@5@+=feaafiart1ev1aaatCvAUfKttLearuWrP9MDH5MBPbIqV92AaeXatLxBI9gBaebbnrfifHhDYfgasaacPC6xNi=xI8qiVKYPFjYdHaVhbbf9v8qqaqFr0xc9vqFj0dXdbba91qpepeI8k8fiI+fsY=rqGqVepae9pg0db9vqaiVgFr0xfr=xfr=xc9adbaqaaeGacaGaaiaabeqaaeqabiWaaaGcbaGaemitaWKaeiikaGccciGae83UdW2aa0baaSqaamXvP5wqSXMqHnxAJn0BKvguHDwzZbqegqvATv2CG4uz3bIuV1wyUbaceaGaa4xmaaqaaiaa+DcaaaGccqGGPaqkcqGH9aqpcqGGOaakcqaIXaqmcqGHsislcqWGLbqzdaahaaWcbeqaaiabgkHiTiab=T7aSnaaDaaameaacaGFXaaabaGaa43jaaaaliabgEna0kabisda0aaakiabcMcaPmaaCaaaleqabaGaeGymaeJaeGimaadaaOGaeiikaGIaemyzau2aaWbaaSqabeaacqGHsislcqWF7oaBdaqhaaadbaGaa4xmaaqaaiaa+DcaaaWccqGHxdaTcqaI0aanaaGccqGGPaqkdaahaaWcbeqaaiabikdaYiabikdaYiabiEda3aaaaaa@5C62@

The MLE of *λ'*_1 _based on the score function was estimated 0.011. The variance of *λ'*_1 _from the inverse of the second derivative of the above likelihood function was estimated as 0.000011. An unconditional variance of *λ'*_2 _via the prevalence pool equation was therefore estimated as 0.000011 × (1114^2^/105^2^). We believe that such an approximation may not be unreasonable because the estimate of *λ'*_1 _using the likelihood function in (B.3) was very close to *λ*_1 _using the joint likelihood of *λ*_1 _and *λ*_2 _in Table 2.

### B.2 The illness-death Markov model

If we assume *λ*_1 _conditionally independent of *λ*_3_(i.e., E(*λ*_1_|*λ*_3_, *λ*_2_) = E(*λ*_1_| *λ*_2_)), the unconditional variance of *λ*_1 _and *λ*_2 _can be calculated as above.

To calculate the unconditional variance of *λ*_3_, we assumed *λ*_3 _was conditionally independent of *λ*_1_. The unconditional variance of *λ*_3 _was:

*Var*(*λ*_3_) = *Var*(*E*(*λ*_3 _| *λ*_2_) + *E*(*Var*(*λ*_3 _| *λ*_2_)

As above, E(Var(*λ*_3_|*λ*_2_)) can be assumed to be equal to the observed Var(*λ*_3_|*λ*_2_), obtained from the inverse of the second derivative of the likelihood function based on MLE estimate of *λ*_1 _conditional on *λ*_2 _and *λ*_3 _(see Table 5). Also, using equation (3),

Var(E(λ3|λ2)=Var(2DP×J×λ2)=(2DP×J)2=(2DP×D)2×1λ24Var(λ2)
 MathType@MTEF@5@5@+=feaafiart1ev1aaatCvAUfKttLearuWrP9MDH5MBPbIqV92AaeXatLxBI9gBaebbnrfifHhDYfgasaacPC6xNi=xI8qiVKYPFjYdHaVhbbf9v8qqaqFr0xc9vqFj0dXdbba91qpepeI8k8fiI+fsY=rqGqVepae9pg0db9vqaiVgFr0xfr=xfr=xc9adbaqaaeGacaGaaiaabeqaaeqabiWaaaGcbaGaemOvayLaemyyaeMaemOCaiNaeiikaGIaemyrauKaeiikaGccciGae83UdW2aaSbaaSqaaiabiodaZaqabaGccqGG8baFcqWF7oaBdaWgaaWcbaGaeGOmaidabeaakiabcMcaPiabg2da9iabdAfawjabdggaHjabdkhaYjabcIcaOKqbaoaalaaabaGaeGOmaiJaemiraqeabaGaemiuaaLaey41aqRaemOsaOKaey41aqRae83UdW2aaSbaaeaacqaIYaGmaeqaaaaakiabcMcaPiabg2da9iabcIcaOKqbaoaalaaabaGaeGOmaiJaemiraqeabaGaemiuaaLaey41aqRaemOsaOeaaOGaeiykaKYaaWbaaSqabeaacqaIYaGmaaGccqGH9aqpcqGGOaakjuaGdaWcaaqaaiabikdaYiabdseaebqaaiabdcfaqjabgEna0kabdseaebaakiabcMcaPmaaCaaaleqabaGaeGOmaidaaOGaey41aqBcfa4aaSaaaeaacqaIXaqmaeaacqWF7oaBdaqhaaqaaiabikdaYaqaaiabisda0aaaaaGccqWGwbGvcqWGHbqycqWGYbGCcqGGOaakcqWF7oaBdaWgaaWcbaGaeGOmaidabeaakiabcMcaPaaa@7311@

A similar procedure was applied to calculate the variance of the regression coefficient *β*, assuming *λ*_21 _independent of *λ*_22_.

## Pre-publication history

The pre-publication history for this paper can be accessed here:


